The article "An Evolutionary Frog Leaping Algorithm for Global Optimization Problems and Applications" was published in 2021. Journal: Comput Intell Neurosci.

# An Evolutionary Frog Leaping Algorithm for Global Optimization Problems and Applications

**DOI:** 10.1155/2021/8928182

**Published:** 2021-12-14

**Authors:** Deyu Tang, Jie Zhao, Jin Yang, Zhen Liu, Yongming Cai

**Affiliations:** ^1^School of Medical Information and Engineering, Guangdong Pharmaceutical University, Guangzhou 510006, China; ^2^School of Computer Science & Engineering, South China University of Technology, Guangzhou 510006, China; ^3^Department of Information Management Engineering, School of Management, Guangdong University of Technology, Guangzhou 510520, China

## Abstract

Shuffled frog leaping algorithm, a novel heuristic method, is inspired by the foraging behavior of the frog population, which has been designed by the shuffled process and the PSO framework. To increase the convergence speed and effectiveness, the currently improved versions are focused on the local search ability in PSO framework, which limited the development of SFLA. Therefore, we first propose a new scheme based on evolutionary strategy, which is accomplished by quantum evolution and eigenvector evolution. In this scheme, the frog leaping rule based on quantum evolution is achieved by two potential wells with the historical information for the local search, and eigenvector evolution is achieved by the eigenvector evolutionary operator for the global search. To test the performance of the proposed approach, the basic benchmark suites, CEC2013 and CEC2014, and a parameter optimization problem of SVM are used to compare 15 well-known algorithms. Experimental results demonstrate that the performance of the proposed algorithm is better than that of the other heuristic algorithms.

## 1. Introduction

In these years, a large number of complex nonlinear optimization problems are solved using mathematical tools by mathematic models. In these cases, traditional approaches often cannot obtain a better solution, which promotes the development of the heuristic optimization techniques. Metaheuristic approach is inspired by the characteristics of the different species in nature, which has rapidly progressed by the theory of biology, physics, society, and so on. Not only one solution but also several solutions are obtained by the heuristic process to find the exact or approximate global optimum. In order to accelerate the convergence speed and find the global solution, researchers have proposed more and more new or improved algorithms. These approaches can be divided into three categories: swarm intelligence (SI), evolutionary algorithms (EAs), and physical phenomena (PP) algorithms.

Swarm intelligence algorithms are inspired by the collective behaviors of natural species such as insects, animals, microorganism, and human. In SI algorithms, the population is a set of individuals (solutions) distributed in search space, which can work in cooperation by survival or competition mechanism to solve problems. In these years, more SI algorithms have been proposed, such as spotted hyena optimizer (SHO) [1], forest optimization algorithm (FOA) [2], particle swarm optimization (PSO) [3], whale optimization algorithm (WOA) [4], artificial bee colony (ABC) algorithm [5], grey wolf optimizer (GWO) [6], grasshopper optimization algorithm (GOA) [7], teaching-learning-based optimization (TLBO) [8], invasive tumor growth optimization (ITGO) algorithm [9], artificial algae algorithm (AAA) [10], and Salp swarm algorithm [11].

The article "An Evolutionary Frog Leaping Algorithm for Global Optimization Problems and Applications" was published in 2021. Journal: Comput Intell Neurosci.

Evolutionary algorithms (EAs) are inspired by the Darwinian principles of nature's capability to evolve living beings well adapted to their environment. The key is to imitate the individual's evolution through mutation, selection, and crossover operation, thus resulting in a better solution. The typical evolutionary algorithms are genetic algorithms [12, 13], evolutionary strategies [14, 15], evolutionary programming [16], and genetic programming [17]. Fusing the mutation mechanism of PSO, differential evolution (DE) and its improved versions are proposed and have achieved greater success in many fields for the continuous optimization problems, such as the typical differential evolution (DE) [18] and adaptive differential evolution (SHADE, LSHADE, and iL-SHADE) [19–21].

Physical phenomena (PP) algorithms mimic physical rules in some physical phenomena. Contrast to SIs or EAs, each individual in a population moves and communicates in the search space according to the physical rules. The typical PP algorithms are thermal exchange optimization (TEO) [22], gravitational search algorithm (GSA) [23], lightning attachment procedure optimization (LAPO) [24], black hole (BH) [25], ray optimization (RO) algorithm [26], and so on.

In recent decades, more than hundreds of population-based optimization algorithms have been proposed yet. We are puzzled: is it necessary to propose a new or improved optimization algorithm? Fortunately, the No Free Lunch (NFL) theorem [27] has been proposed. This theorem has logically proved that there is no metaheuristic algorithm best suited for solving all the optimization problems. It is to say that a particular metaheuristic approach may show very good results on a set of problems, but the same algorithm may show poor performance on a different set of problems. Therefore, we need to propose a new approach to solve the continuous optimization problems, which can better achieve the balance between the exploitation ability and the exploration ability. In addition, we want that the proposed method can solve more different optimization problems whether they are in the coordinate system or in the rotated coordinate system. In this paper, we focus on the research about the advantages and disadvantages of the shuffled frog leaping algorithm (SFLA) [28] and the related technique in order to propose a new approach for the continuous optimization problems.

The article "An Evolutionary Frog Leaping Algorithm for Global Optimization Problems and Applications" was published in 2021. Journal: Comput Intell Neurosci.

The shuffled frog leaping algorithm is a SI algorithm inspired by the foraging behavior of frogs, which combines the mechanism of meme diffusion for the global exploration and search by PSO for the local exploitation. Due to its simplicity and efficiency, it has been widely applied to many real-world optimization problems such as the traveling salesman problem (TSP) [28], vehicle routing problem [29], economic dispatch problem [30, 31], 0/1 knapsack problem [32], resource-constrained project scheduling problem [33, 34], flow shop scheduling problem [35, 36], and grid task scheduling problem [37]. The version of SFLA for the discrete optimization problems has achieved great success, but the version of SFLA for the continuous optimization problems is not performing well due to its low convergence speed and premature problem. In this case, some improved versions of SFLA have been proposed. For instance, Xia Li et al. [38] considered the historical information for the local exploration and proposed an extremal optimization process, which was completed by the fine-grained Gaussian mutation and the coarse-grained Cauchy mutation. In order to enhance the diversity of population and the local exploration ability, the opposition-based learning (OBL) strategy was used in literature [39]. The initial population was produced by the basic uniform distribution and the opposition-based learning process, which reinforces the diversity of the population. In addition, the frog leaping rule was improved by the normal and opposition-based search. Morteza Alinia Ahandani et al. [40] diversified the search rule of SFAL by the differential evolution operator substituted for the basic frog leaping rule. Sharma S et al. [41] found that it was not enough that each worst frog was guided only by the best frog in each subpopulation. So, the centroid of three new individuals was considered for the frog leaping rule. Hong-bo Wang et al. [42] combined the historical information, information of the local frog and global frog substituted for the basic frog leaping search method, and the mutation operation by the normal distribution and Cauchy distribution was used for the globally best frog and the worst frog. Liu C et al. [43] used the chaotic opposition-based learning to achieve the population initialization, and then the adaptive nonlinear inertia weight and the perturbation operator strategy based on Gaussian mutation were used for the balance between the exploration and the exploitation. Paper [44] presents grouped SFLA for solving continuous optimization problems combined with the excellent characteristics of cloud model transformation between qualitative and quantitative research. Deyu Tang et al. [45] proposed a lévy flight mutation operator for the frog leaping rule and an interaction learning rule for the global search. Wenjuan Li et al. [46] used quantum movement equations to search for the optimal location according to the co-evolution of the quantum frog colony.

The article "An Evolutionary Frog Leaping Algorithm for Global Optimization Problems and Applications" was published in 2021. Journal: Comput Intell Neurosci.

As mentioned above, we find that the shuffled frog leaping algorithm has been successfully applied to many combinatorial optimization problems, but it is not efficient for the continuous optimization problem due to the weakness of balance between the exploration and the exploitation, such as the weakness of the exploitation ability (the local search ability) and the loss of the exploration operator (the global search operator). Only using the shuffled strategy and the guidance by the best local frog is not enough for the complex problems such as the multimodal optimization problems. Therefore, researchers used the opposition-based learning strategy [39], chaotic strategy [43], and so on to enhance the diversity of the population. Meanwhile, the differential operators [40] and the reserving the historical information strategy [38] are adopted for the exploration. In addition, the first version of quantum inspired SFLA by Q-bits and Q-gate [46] was proposed, which can be seen as the quantum computing approach. However, the quantum simulation approach has not been utilized for SFLA. So far, the improved versions of SFLA are still based on the PSO framework. In addition, we find that some improved SFLA algorithms can be used successfully to solve the optimization problems in the coordinate system but lose to solve these problems in the rotated coordinate system or contrary. Therefore, we attempt to establish a new framework of SFLA based on quantum evolution and eigenvector evolution in order to achieve the balance between the exploitation (quantum evolution) and the exploration (eigenvector evolution) to solve more different optimization problems whether they are in the coordinate system or in the rotated coordinate system.

The major contributions are as follows. First, we propose a two-stage search framework of SFLA based on the quantum evolution and eigenvector evolution for the balance between the exploitation and the exploration. Second, the exploitation is achieved by a quantum evolutionary operator with historical information for the frog leaping rule. Third, the exploration is achieved by the adaptive eigenvector evolutionary operator.

The article "An Evolutionary Frog Leaping Algorithm for Global Optimization Problems and Applications" was published in 2021. Journal: Comput Intell Neurosci.

The rest of the paper is organized as follows. In Section 2, the shuffled frog leaping algorithm is introduced. Related work is reviewed and discussed in Section 3. In Section 4, we propose the evolutionary frog leaping algorithm. Experimental results and analysis are shown in Section 5. Finally, conclusions and further discussions are given in Section 6.

## 2. Shuffled Frog Leaping Algorithm (SFLA)

The shuffled frog leaping algorithm is a heuristic approach inspired by the frog foraging behavior, which is designed according to the memetic evolution principle and the PSO framework. Suppose each frog has thought and is living by the meme information (culture information). The frog population is divided into different memeplexes (communities or groups) according to the common thought (or meme). In each global iteration step, memeplexes are divided again by the shuffled process according to the memetic evolution principle, which can be seen as the global exploration process. In each submemeplex, the frog leaping process is achieved by the simplified PSO, which can be seen as the local exploration process. In each local step, the worst frog and the best frog are obtained, and the worst frog is guided by the best frog to find the best food. The memetic evolution process and the frog leaping process are completed alternately corresponding to the balance between the exploration and the exploitation. The SFLA can be described as follows: Firstly, the initial population is generated randomly and divided into *m* submemeplexes in a descending sort. The shuffled process can be represented as equation (1) where popsize (popsize=*m* × *n*) is an integer which indicates the population size, *m* indicates the number of memeplexes, and *n* indicates the number of frogs in each submemeplex. The fitness *f*(*i*) for the *i*th frog can be evaluated and sorted in descending order to form *m* memeplexes *H*^*1*^*H*^2^,…, *H*^*b*^,…, *H*^m^, which can be constructed by

(1) $$\begin{array}{c} H^{b}=\left\{X_{i}^{b}|X_{i}^{b}=X_{b+m\left(k-1\right)},k=1,2,\ldots ,n\right\},\;b=1,2,\ldots ,m, \end{array}$$

where *H* is a set of solutions in a memeplex and *X*_*i*_ indicates a solution and it is a vector.

Second, the frogs finish the updating step in each submemeplex according to the following equation:

(2) $$\begin{array}{c} X_{\text{worst}}^{\prime }=X_{\text{worst}}+\text{rand}\cdot \left(X_{\text{best}}-X_{\text{worst}}\right), \end{array}$$

where *X*_worst_ represents the position of the worst frog, *X*_best_ represents the position of the best frog, *ran*  *d* denotes a random number of uniform distribution between (0, 1), and *X*_worst_ and *X*_best_ belong to the same submemeplex. If the fitness of *X*_worst_′ is better than *X*_worst_, *X*_worst_ is updated. Otherwise, *X*_best_ is replaced by the position of the globally best frog *X*_*g*_; if the fitness of *X*_worst_′ is better than *X*_worst_, *X*_worst_ is updated. If there is still no improvement, a feasible solution is generated to replace *X*_worst_. This updating step can be seen as a local search step, which continues until the threshold value reaches the predefined number of iteration within each memeplex. The local search step and the shuffling processes alternate until a predefined convergence criterion is satisfied. The time complexity of getting the best frog and the worst frog in a submemeplex is *O*(*n*), where *n* is the number of frogs in each submemeplex. Thus, the total time complexity of SFLA is as follows:

(3) $$\begin{array}{c} O\left(\text{SFLA}\right)=O\left(m*k*n*T*D\right)=O\left(ps*k*T*D\right), \end{array}$$

where *ps* is the population size, *m* is the number of submemeplexes, *k* is the local iteration number in each submemeplex, *n* is the number of frogs in each submemeplex, *ps*=*m∗n*, *T* is the number of the total iteration, and *D* is the dimension. Pseudo code of SFLA is shown in Algorithm 1.

The article "An Evolutionary Frog Leaping Algorithm for Global Optimization Problems and Applications" was published in 2021. Journal: Comput Intell Neurosci.

## 3. Related Research

The balance between the exploitation and the exploration is a core task for metaheuristic approach. For this goal, some approaches use one operator with more units to achieve this task, such as PSO. The search operator of PSO is accomplished by the global search unit and historical search unit, in which the global search unit achieves the exploitation task and historical search unit achieves the exploration task. Another approach uses two or more operators to achieve the balance between the exploitation and the exploration, such as ABC, CS, and TLBO. For the ABC, the operator of employed bees and the operator of scout bees achieve exploration task and the operator of onlooker bees achieves exploitation task. For the CS, lévy flight operator achieves exploitation task with a mutation method and nest selection operator achieves the exploration task. For TLBO, the teaching operator achieves the exploitation task and the learning operator achieves the exploration task. As we know, the SFLA has only one operator, which achieves the exploitation task. The operator for exploration of SFLA is missing. Therefore, the framework by the two stage for SFLA can be considered.

### 3.1. Quantum Simulation (QS) Methods

In 2004, J. Sun et al. [47] proposed the first quantum behaved particle swarm optimization, which simulates the quantum evolutionary process under the particle swarm optimization framework. After that, many improved QS algorithms are developed such as weighed mean best position [48], Gaussian probability distribution for the local attractor [49], group search optimizer [50], diversity control strategy [51, 52], cooperative mechanism [53], chaotic mutation operator [54], decentralized strategy with cellular structured population [55], memetic algorithm [56], two-stage search method [57], and collaborative attractor [58]. More and more improved versions of QPSO are based on the basic quantum simulation model. The quantum search operator is proposed according to the Schrodinger equation and Monte Carlo method.

The article "An Evolutionary Frog Leaping Algorithm for Global Optimization Problems and Applications" was published in 2021. Journal: Comput Intell Neurosci.

The state function $\psi \left(\bar{x},t\right)$ in time can be represented by the Schrodinger equation, in which $\hat{H}$ is the Hamiltonian operator and *t* denotes the time.

(4) $$\begin{array}{c} ih\frac{\partial }{\partial t}\psi \left(\bar{x},t\right)=\hat{H}\psi \left(\bar{x},t\right). \end{array}$$

The mass *m* of one particle in a potential field $V\left(\bar{x}\right)$ can be represented as follows:

(5) $$\begin{array}{c} \hat{H}=-\frac{h^{2}}{2m}\nabla^{2}+V\left(\bar{x}\right), \end{array}$$

where *h* means the Planck constant.

Using the Monte Carlo method, we can obtain equation (6) according to the Delta potential well model:

(6) $$\begin{array}{c} X_{i}=P_{i}\pm g\left|X_{i}-P_{i}\right|\ln\left(\frac{1}{\text{rand}}\right), \end{array}$$

where *g* denotes the parameter of search, *P*_*i*_ is the potential well, *X*_*i*_ denotes a particle *i* in *D* dimensional space, and rand denotes a random number of uniform distribution between (0, 1).

Considering the convergence, *X*_*i*_(*t*)⟶*P*_*i*_(*t*), when *t*⟶*∞*. Here, *t* denotes the time. Quantum simulations have not been used for SFLA, so we attempt to achieve the quantum evolution as a component of SFLA for the exploitation.

### 3.2. Eigenvector Approach

Eigenvector information of the covariance matrix of a set can rotate the coordinate system, and it can be used for a multivariate statistical method of principal component analysis (PCA) [59], which can reduce the dimension of the handled multivariate data to some extent. The inspiration of PCPSO is derived from a methodology known as the Lagrange point of view [60] for creating and flying in a dynamic coordinate system with the particles. Chu et al. [61] introduced principal component analysis into PSO to remedy the problem caused by the absorbing bound-handling approach. Inspired by the Hamiltonian Monte Carlo (HMC) method, Kuznetsova et al. [62] proposed the PCA-based stochastic optimization (PCA-SO) algorithm. Xinchao Zhao et al. [63] proposed the improved version of PSO by the PCA and the line search method. All these approaches are based on the principle of PCA, in which eigenvector has not been used directly for the optimization problem. In 2015, literature [64] first proposed an eigenvector-based crossover operator for differential evolution (DE) in order to improve the performance of nonrotationally invariant crossovers by rotating the coordinate system to make the function landscape be pseudo-separable. In 2016, Noor H. Awad et al. [65] used the eigenvector-based crossover operator and other methods to improve the LSHADE version and proposed the LSHADE-EpSin algorithm. However, the eigenvector search method is sensitive to the parameter setting. In this paper, we attempt to achieve a simple eigenvector evolutionary operator without parameter setting as a component of SFLA for the exploration.

The article "An Evolutionary Frog Leaping Algorithm for Global Optimization Problems and Applications" was published in 2021. Journal: Comput Intell Neurosci.

To sum up, the SFLA has the idea of balance between the exploitation and the exploration. However, the exploitation by frog leaping rule is only guided by the best frogs, which can speed up the convergence but is easy to fall into the local optimum. More importantly, the real exploration operator in SFLA is missing. In quantum simulation approach, the individual is guided by the potential well not the best individual, which can enhance the diversity of population. So, it can be considered as the component of SFLA for exploitation. The eigenvector crossover operator has achieved the rotationally invariant of differential evolution for complex optimization problems. However, the real eigenvector search approach without parameter setting is not proposed. If an eigenvector evolutionary operator can be completed, it can be considered as the component of SFLA for the exploration operator.

## 4. The Proposed Approach

In SFLA, frogs only have jumping behavior to spread information like humans, which is not enough to simulate their social behaviors. Indeed, interactive learning among a population is popular in society. Therefore, interactive learning characteristic can be modeled to simulate the social behaviors of frogs. In this paper, we propose a two-stage search framework of SFLA for the balance between the exploitation and the exploration. In the first search stage, the local search is achieved in terms of the quantum evolutionary operator instead of the PSO operator, which simulates the jumping behavior of frogs in the quantum space. In the second search stage, the global search is achieved in terms of the adaptive eigenvector evolutionary operator instead of only using the shuffled operator, which simulates the interactive learning characteristic of frogs.

The article "An Evolutionary Frog Leaping Algorithm for Global Optimization Problems and Applications" was published in 2021. Journal: Comput Intell Neurosci.

### 4.1. Quantum Evolutionary Operator

The quantum evolutionary operator is achieved in different submemeplexes by the shuffled process as equation (1). Therefore, it can be considered as a local search process. According to the quantum simulation model introduced above, we know that the quantum evolutionary operator is achieved by the Monte Carlo method according to the potential well model. In equation (6), considering the convergence, *X*_*i*_(*t*)⟶*P*_*i*_(*t*), when *t*⟶*∞*, where *P*_*i*_ is considered as the potential well. The basic quantum evolutionary operator only uses one potential well, which accelerates the search speed but is easy to fall into the local optimum. For this, we propose the second potential well with memory to enhance the search ability for quantum evolution. The new search operator can be represented by the following equation.

(7) $$\begin{array}{c} X_{i}=P_{i}\pm g.\left|X_{i}-P_{i}^{\prime \text{memory}}\right|\ln\left(\frac{1}{\text{rand}}\right),\;i=1,2,\ldots ,\text{popsize}, \end{array}$$

where *P*_*i*_ denotes the first potential well, *P*_*i*_^′memory^ denotes the second potential well, *g* is the search parameter, and popsize is the population size. rand denotes a random number of the uniform distribution in [0, 1]. *P*_*i*_ is a vector in *D* dimensional space, and *P*_*i*_^′memory^ is also a vector in *D* dimensional space.

In SFLA, the frog leaping rule equation (2) can be considered as the first potential well *P*_*k*_ because the location of the search is located in a rectangle area between the worst frog and the best frog. It can be represented as the following equation:

(8) $$\begin{array}{c} P_{i}=X_{\text{worst}}+\text{rand}\cdot \left(X_{\text{best}}-X_{\text{worst}}\right)=w\cdot X_{\text{worst}}+\left(1-w\right)\cdot X_{\text{best}},w=\text{rand}\cdot \left(0,1\right),\;i=1,2,\ldots ,\text{popsize.} \end{array}$$

The second potential well can be represented by equations (9) and (10).

(9) $$\begin{array}{c} P_{i}^{\prime }=\frac{1}{n}\overset{n}{\underset{c=1}{\sum }}X_{c}, \end{array}$$

where *P*_*i*_′ indicates the means of *n* positions of frogs in a submemeplex (a group), and it is a local center.

(10) $$\begin{array}{c} P_{i}^{\prime \text{memory}}=\frac{P_{i}^{\prime \text{memory}}}{v}+P_{i}^{\prime }. \end{array}$$

Equation (10) denotes a recurrence formula, *v* is an integer, and it is increased from 1 to *n*(*v*=1,2,…, *n*). The initial value of *v* is set as 1. *n* is the number of frogs in a submemeplex, which is equal to the iteration number of the local search process. The initial *P*_*i*_^′memory^ is a zero vector.

(11) $$\begin{array}{c} g=1\text{.}5-\text{0.}5*\frac{\text{FES}}{\text{MAX\_FES}}\text{.} \end{array}$$

Equation (11) is a linear function, which controls the search scope. FES is the fitness evaluation number, and MAX_FES is the max numbers of fitness value.

The article "An Evolutionary Frog Leaping Algorithm for Global Optimization Problems and Applications" was published in 2021. Journal: Comput Intell Neurosci.

Figure 1 shows an instance of the quantum evolutionary process. First, the population is divided into different submemeplexes according to equation (1). It can be observed in the left section of Figure 1. Twelve frogs in the population are divided into three submemeplexes (different colors such as green, yellow, and purple), and there are four frogs in each submemeplex. The 12 frogs *X*_1_, *X*_2_, *X*_3_, .., *X*_12_ are arranged according to the descending order by fitness value. For example, *X*_6_ is an ordinary frog, it can be arranged into the purple submemeplex according to equation (1), i.e., *X*_6_ = *X*3 + 3 *∗* (2 − 1) (*b* = 3, *k* = 2). *X*_3_ denotes the best frog, and *X*_12_ denotes the worst frog in the purple submemeplex. The quantum evolution operator is achieved by the worst frog in each submemeplex. The search process can be observed in the search space (the right section of Figure 1). The 12 balls in search space are corresponding to the 12 rectangles in fitness space for 12 frogs. The red ball with vertical line denotes the first potential well *P*_*i*_, the blue ball with horizontal line denotes the second potential well *P*_*i*_′, and the grey ball with horizontal line denotes the historical *P*_*i*_′. *P*_*i*_^′memory^ is achieved by the current *P*_*i*_′ (blue ball) and the historical *P*_*i*_′ (grey ball) by the recurrence formula in equation (10). The first potential well *P*_*i*_ is obtained in a rectangle region by a diagonal between *X*_worst_ and *X*_best_ according to equation (8). In fact, it is the basic search operator of the shuffled frog leaping algorithm. The worst frog *X*_worst_ runs toward the position of the best frog *X*_best_, and it is easy to converge to the local optimum. Fortunately, the worst frog *X*_worst_ is guided not only by the first potential well *P*_*i*_ but also by the second potential well *P*_*i*_′ in the quantum evolutionary operator. The basic second potential well *P*_*i*_′ is the centroid of the local submemeplex according to equation (9). It can be observed that *P*_*i*_′ can guide the worst frog *X*_worst_ search in a quadrilateral region by the frog *X*_3_, *X*_6_, *X*_9_, and *X*_12_ as shown in Figure 1, which can enhance the diversity of the population. However, it cannot ensure that the worst frog *X*_worst_ flees from the local optimum. Therefore, we propose an improved potential well *P*_*i*_^′memory^ instead of *P*_*i*_′, which retains the historical information for each search process. The potential well *P*_*i*_^′memory^ is produced by many historical *P*_*i*_′ (grey balls) and the current *P*_*i*_′ (blue ball), which can ensure that it can run out of the quadrilateral region (it can be seen as equation (10) and Figure 1). It can be observed that the search of the worst frog *X*_worst_ is guided by the first potential well *P*_*i*_ and the second potential well *P*_*i*_^′memory^. In contrast to the old search rule as equation (2), the worst frog *X*_worst_ is not easy to fall into the local optimum (blue region). In other words, the worst frog *X*_worst_ has more opportunities to run toward the direction of the global optimum (red region) guided by the different potential wells not only guided by the best frog X_best_.

The article "An Evolutionary Frog Leaping Algorithm for Global Optimization Problems and Applications" was published in 2021. Journal: Comput Intell Neurosci.

### 4.2. Adaptive Eigenvector Evolutionary Operator

Interactive learning behavior is achieved in the whole population not in the local population (a submemeplex). Therefore, it is a global search process. It can be represented as the following equation:

(12) $$\begin{array}{c} Y_{i}=X_{i}+2\cdot \text{rand}\cdot \left(X_{v}-X_{o}\right), \end{array}$$

where *X*_*i*_, *X*_*v*_,  and *X*_*o*_ are three vectors in *D* dimensional space corresponding to three frogs. *i*, *v*,  and *o*(*i* ≠ *v* ≠ *o*) are three different integers in a set as {1,2,…popsize}, where popsize is the population size. *X*_*i*_ is a solution vector, which can be updated by the difference between *X*_*v*_ and *X*_*o*_. rand denotes a random number of the uniform distribution in [0, 1]. $\bar{X_{i,*}}$ is the mean of all the *X*_*i*_ in the population, and $\bar{X_{j,*}}$ is the mean of all the *X*_*j*_ in the population.

(13) $$\begin{array}{c} \mathrm{cov}\left(i,j\right)=\frac{\sum_{k=1}^{\text{popsize}}\left(X_{i,k}-\bar{X_{i,*}}\right)\left(X_{j,k}-\bar{X_{j,*}}\right)}{\text{popsize}-1}. \end{array}$$

To compute the eigenvector basis, we factorize the covariance matrix cov(*Y*) into a canonical form as follows:

(14) $$\begin{array}{c} \mathrm{cov}\left(X\right)=Q\Lambda Q^{-1}, \end{array}$$

where *Q* is the square matrix (*D* rows and *D* columns) whose *i*_*th*_ column is the eigenvector *q*_*i*_ of cov(*Y*). Λ is the diagonal matrix whose diagonal elements are the corresponding eigenvalues. The eigenvector evolutionary operator can be represented as follows:

(15) $$\begin{array}{c} Y_{i,j}^{\prime }=\left\{\begin{array}{cc} {\left[Q^{T}\cdot X_{i}\right]}_{j}, & j\notin U_{i},\\ {\left[Q^{T}\cdot Y_{i}\right]}_{j}, & j\in U_{i}, \end{array}\right.\;i=1,2,\ldots ,\text{popsize};j=1,2,\ldots D, \end{array}$$

where *X*_*i*_ (or *Y*_*i*_) denotes an individual and it is a vector with one column and *D* rows, *Q*^*T*^ is a square matrix by *D* rows and *D* columns, and *D* denotes the dimension of a solution vector. So, [*Q*^*T*^ · *X*_*i*_] (or[*Q*^*T*^ · *Y*_*i*_]) denotes a new individual, and it is a vector with one column and *D* rows. *U*_*i*_ is a set of integers as {1,2, 3,…, *D*}, which denotes the randomly selected *r* rows for the individual ([*Q*^*T*^ · *Y*_*i*_]), and *r* is a randomly selected integer from the set as {1,2, 3,…, *D*}.

(16) $$\begin{array}{c} Y_{i}^{\text{eig}}=Q\cdot Y_{i}^{\prime }. \end{array}$$

When the solution is updated in the eigenvector basis, the updating behavior will become rotationally invariant in the natural basis. To reduce the risk of ineffective behavior of rotationally invariant operator (*Y*^eig^), we introduce an adaptive selection strategy for the original operator and the eigenvector evolutionary operator.

(17) $$\begin{array}{c} X_{i\left(\text{new}\right)}=\left\{\begin{array}{cc} Y_{i}, & \text{IF rand}<p,\\ Y_{i}^{eig} & \text{else,} \end{array}\right. \end{array}$$

where rand is a random number of uniform distribution in [0, 1] and *p* is a self-adapting selection parameter value. It can be represented as follows:

(18) $$\begin{array}{c} p=p*\left(1-\frac{1}{ps_{0}}\right)+\left(\frac{1}{ps_{0}}\right)*\left(\frac{p1}{p1+p2}\right). \end{array}$$

The initial value *p*_0_=0.5 and *ps*_0_=2. *p*1 denotes the number of success by original operator as shown in equation (12), and *p*2 denotes the number of success by eigenvector evolutionary operator as shown in equation (16).

The article "An Evolutionary Frog Leaping Algorithm for Global Optimization Problems and Applications" was published in 2021. Journal: Comput Intell Neurosci.

Here, we explain our approach by a shifted rotated expanded Scaffer F6 function in a two-dimensional space (shown in Figures 2 and 3).  Figure 3 shows the major characteristic of the eigenvector basis, and the eigenvector evolution shows the search direction in a rotationally invariant. Considering the complexity of real-world optimization problems, the original operator and the eigenvector evolutionary operator are running alternately according to the success rate, and it is achieved by an adaptive selection mechanism (equations (17) and (18)). Pseudo code of the proposed approach is shown in Algorithm 2.

## 5. Experimental Results and Analysis

To test the performance of the proposed approach, we conduct a real-world parameter optimization problem of SVM and the 30 benchmark functions recommended by literature [45], CEC2013 [66], and CEC2014 [67]. Fifteen functions (F1–F15) belong to the basic optimization problem, nine functions (F16–F24) belong to CEC2013, and six functions (F25–F30) belong to CEC2014. Different problems (unimodal, multimodal, rotated, and composition) are considered. To verify the effectiveness of the proposed algorithm, 12 well-known algorithms including NNA [68], LAPO [69], GbABC [70], SFLA [71], SCA [72], SSA [11], GWO [6], CMAES [73], WQPSO [48], TSQPSO [57], SaDE [74], and AAA [10] are used for benchmark suites. Each algorithm is carried out independently on the same machine by the MATLAB 2009R for 30 runs. For fair comparison, the fitness evaluation number (FES) is used instead of using the number of iteration. The max evaluation number (MAX_FES) is set as *D∗*1*E*4, and *D* is the dimension. We record all the fitness evaluations and the error values (*f*(*x*) − *f*(*∗*)), where *f*(*∗*) denotes the global optimum value. The basis analysis such as mean and standard deviation is used. In addition, we adopt the *T*-test [75], Wilcoxon signed-rank test [76], and Friedman test [76].

The article "An Evolutionary Frog Leaping Algorithm for Global Optimization Problems and Applications" was published in 2021. Journal: Comput Intell Neurosci.

Wilcoxon's test is used in our experimental study, the first step is to compute the *R* + and R− related to the comparisons between EFLA and the rest of algorithms. Let *R* + be the sum of ranks for the problems in which the first algorithm outperformed the second, and R− be the sum of ranks for the opposite. Once they have been obtained, their associated *p* values can be computed. The null hypothesis H0 was used for the Wilcoxon signed-rank tests for purpose of this paper. The statistical significant value used to test H0 hypothesis is *τ* = 0.05. If in any test a *p* value that is smaller than or equal to significance level *τ* value is produced, then the H0 hypothesis for that test is rejected and the alternative hypothesis is selected.

The Friedman test is a nonparametric analog of the parametric two-way analysis of variance, which can be used to detect whether there exist significance among the results of the algorithms. Inside the field of statistics, hypothesis testing can be used to draw inferences about one or more populations from the given results. The null hypothesis for Friedman's test states equality of results between the algorithms. The alternative hypothesis is defined as the negation of the null hypothesis, so it is nondirectional. The statistical significance value used to test H0 hypothesis is *τ* = 0.05. If in any test a *p* value that is smaller than or equal to significance level *τ* value is produced, then the H0 hypothesis for that test is rejected and the alternative hypothesis is selected. It ranks the algorithms for each problem separately; the best performing algorithm ranks 1, the second best has a rank of 2, and so on.

The details of the 30 benchmark functions are shown in Table 1, and the parameter setting of 13 algorithms is shown in Table 2.

The article "An Evolutionary Frog Leaping Algorithm for Global Optimization Problems and Applications" was published in 2021. Journal: Comput Intell Neurosci.

### 5.1. Experimental Results and Analysis on the First Test Suite for Low Dimension (*D* = 30)

In this test, we compare the proposed algorithm with the 12 well-known algorithms for the 30 benchmark functions in low dimension (*D* = 30). Tables 3 and 4 show the comparison results with EFLA and 12 algorithms including two quantum simulation based-PSO versions (TSQPSO and WQPSO), seven SI algorithms (NNA, LAPO, SFLA, SSA, SCA, GWO, and AAA), an improved ABC algorithm (GbABC), and two evolutionary algorithms (SaDE and CMAES). The mean and standard deviation of the error values obtained by the 13 algorithms are listed in Tables 3 and 4, where the performance rank of the 13 algorithms is also represented. The character ‘R' in the first line of Tables 3 and 4 is the abbreviation of word ‘rank'; each column starting with ‘R' after each algorithm denotes the rank of the 13 algorithms. It can be observed that the proposed algorithm is a competitive SFLA variant for the first test suite. According to the theorem of ‘No Free Lunch' [27], one algorithm cannot offer better performance than all the others on every aspect or on every kind of problem. This is also observed in our experimental results. In optimizing the 30 functions, EFLA is ranked the first for 10 times, the second for 7 times, the third for 5 times, and ranked the fourth and fifth for 2 and 1 times, respectively. Compared with the solution accuracy on seven unimodal functions (F1, F2, F3, F4, F16, F17, and F18), EFLA is ranked first 2 times, CMAES is ranked first 2 times, SaDE is ranked first 2 times, LAPO is ranked first 4 times, SaDE and EFLA are ranked first 2 times, and GWO is ranked first 1 time. It indicates that EFLA achieves the global optimum for sphere function (F1) and Schwefel's problem 1.2 (F3). On many multimodal functions, EFLA represents the better exploration ability than others. Rastrigrin function (F5) and Griewank function (F7) have many local optima, and it can be seen that EFLA obtains the global optimum. Especially, it is observed that EFLA achieves better solution accuracy than the other 12 algorithms for the hybrid function 1 (*N* = 3) and hybrid function 2 (*N* = 3), which are complex multimodal and nonseparable problems. We can also observe that EFLA achieves the better solution accuracy than LAPO TSQPSO, WQPSO, GbABC, NNA, SaDE, SFLA, SSA, CMAES, SCA, AAA, and GWO for F1, F3, F5, F7, F10, F11, F23, F26, F27, and F29.

For the thorough analysis, the ‘robustness' in this paper is used to evaluate the search stability of the algorithms under different condition (such as the rotated and unrotated test function). It means that the proposed algorithm can obtain better performance whether the optimization problem is in the rotated system or in the unrotated system. We know that the 30 optimization problems in this suite are combined by the two types. Type 1 (F1–F15) is the basic unrotated benchmark functions, and Type 2 (F16–F30) is the rotated, composition or hybrid problems. It is observed from Tables 3 and 4 that WQPSO, CMAES, SaDE, and SSA can achieve the better solution accuracy for Type 2 but poor accuracy for Type 1. Contrary, LAPO, SCA, NNA, TSQPSO, GbABC, and GWO can achieve the better accuracy for Type 1 but poor accuracy for Type 2. In comparison with them, it is observed that EFLA achieves the better solution accuracy for more optimization problems including not only Type 1 but also Type 2, which means that it has the better robustness than others.

The article "An Evolutionary Frog Leaping Algorithm for Global Optimization Problems and Applications" was published in 2021. Journal: Comput Intell Neurosci.

The *T*−test method is used to compare the difference between EFLA to the other 12 algorithms for the 30 optimization problems. In these experiments, a two-tailed test with significance level of 0.05 is adopted, and the *p* value and *t*-value are recorded and shown in Tables 5 and 6. The better results of EFLA than other algorithms are shown in bold. ‘−' means that EFLA and the other algorithm obtain almost the same global optimum (it cannot be computed by *t*−test). The last lines in Table 5 and 6 denote the number of ‘B,” ‘N,' and ‘W.' ‘B' means that EFLA is significantly better than the other algorithm, ‘N' means that there is no significant difference between EFLA and the other algorithm, and ‘W' means that the other algorithm is significantly better than EFLA. The average excellent rate between EFLA and the other 12 algorithms for the 30 functions is 71.11%, which can be computed as the following equation:

(19) $$\begin{array}{c} \text{rate}=\frac{\sum_{i=1}^{12}\sum_{j=1}^{30}\left(B_{i,j}\right)}{\sum_{i=1}^{12}\sum_{j=1}^{30}\left(B_{i,j}+N_{i,j}+W_{i,j}\right)}. \end{array}$$

It means the average performance of EFLA is good although it is not always the best for all the functions with respect to the 12 algorithms.

Table 7 indicates more details of comparison results by Wilcoxon's test. ‘+' means that the EFLA is better than the other algorithms.‘ = ' means that the EFLA obtains the equal results than the other algorithms. ‘−' means that the EFLA is less than the other algorithms. The last three columns show the number of winner (*w*), equal (*e*), and lose (*l*) including the *p* values and the *z*-values. Table 7 shows that the average excellent rate between EFLA and the other 12 algorithms for the 30 functions is 80.55%, which can be computed as follows:

(20) $$\begin{array}{c} \text{rate}=\frac{\sum_{i=1}^{12}\sum_{j=1}^{30}\left(w_{i,j}\right)}{\sum_{i=1}^{12}\sum_{j=1}^{30}\left(w_{i,j}+e_{i,j}+l_{i,j}\right)}. \end{array}$$

In addition, Friedman's test is used.  Table 8 shows the average rank of 13 algorithms. We can see that the performance of EFLA is better than that of the other 12 algorithms with the minimal average rank value (3.12).  Table 9 shows that the comparison of 13 algorithms has significant difference with *p* value = 9.43*E* − 11 (<0.05).

The article "An Evolutionary Frog Leaping Algorithm for Global Optimization Problems and Applications" was published in 2021. Journal: Comput Intell Neurosci.

To compare the convergence speed of 13 algorithms, the convergence curve is drawn in Figure 4. We can see that the EFLA outperforms the 12 algorithms for the 6 different optimization problems including unrotated multimodal functions (F3, F7, and F11) and rotated multimodal functions (F23, F27, and F29). It is observed that the proposed algorithm converges faster than the others in overall iteration process for F7, F28, and F29. For rotated Schwefel's function (F23), SSA converges faster than EFLA in the early iteration. However, in the late iteration, EFLA achieves the best solution than SSA. It means that SSA has the stronger exploitation ability but weak exploration ability. For EFLA, it completes the better balance between exploitation and exploration.

### 5.2. Scalability Analysis for the Second Test Suite for High Dimension (D-100)

We know that the performance of many heuristic optimization algorithms decreases drastically with the increase in the problem scale. In this experiment, we conduct scalability analysis for the 13 algorithms to test the performance of 100-D functions including two unrotated multimodal functions (F1 and F3) and four rotated multimodal functions (F20, F23, F28, and F29). Experimental settings are the same as those described in Table 2.  Table 10 reports the mean and standard deviation of the error values obtained by the 13 algorithms, where the best results are marked in bold. The character ‘**R**' in the first line of Table 10 is the abbreviation of word ‘rank'; each column starting with ‘**R**' after each algorithm denotes the rank of the 13 algorithms. The grey shading of each cell denotes that the performance of EFLA is better than that of the other algorithm. It can be observed that EFLA is ranked the first for 1 times, the second for 2 times, and the third for 3 times, respectively. There are at least four optimization problems that EFLA outperforms each one in the other 12 algorithms. For hybrid function 4 (*N* = 4) (F28), EFLA obtains the better accuracy than LAPO, TSQPSO, WQPSO, GbABC, NNA, SaDE, SFLA, SSA, CMAES, SCA, AAA, and GWO. For sphere function (F1), EFLA obtains the better accuracy than LAPO, TSQPSO, WQPSO, GbABC, NNA, SaDE, SFLA, SSA, CMAES, SCA, and AAA except for GWO.

Particularly, for the multimodal functions, the number of local optima increases drastically with the problem dimension, which makes some algorithms vulnerable to premature convergence. As shown in Table 3, Table 4, and Table 10, EFLA is the robust algorithm that can maintain a good global search ability in such cases for rotated Schwefel's function (F23) and hybrid function 4 (*N* = 5) (F29), whereas the performance of the other algorithms deteriorates severely.  Figure 5 shows the convergence curve of 13 algorithms for the F28 and F29. We can see that EFLA converges faster than 12 algorithms for F23 except F29. Though EFLA converges slowly than some other algorithms such as LAPO and GbABC, for F23, it achieves the best or almost the same fitness value than the other algorithms in the last iteration.

The article "An Evolutionary Frog Leaping Algorithm for Global Optimization Problems and Applications" was published in 2021. Journal: Comput Intell Neurosci.

In addition, Friedman's test is used.  Table 11 shows the average rank of 13 algorithms. We can see that the performance of EFLA is better than that of the other 12 algorithms with the minimal average rank value (2.50).  Table 12 shows that the comparison of 13 algorithms has significant difference with *p* value = 0.001 (< 0.05).

### 5.3. Parameter Sensitivity Analysis

Three parameters in our proposed approach, namely, *popsize, m*, and *n*, should be tuned. *m* is the number of submemeplexes and *n* is the number of frogs in each submemeplex. It is obvious that population size (popsize) is equal to *m∗n*. There are 12 combinations for the three parameters (popsize, *m*, and *n*). The proposed algorithms with 12 different parameter settings are run 30 times for the 30 benchmark optimization problems in Table 13. The results are shown in Table 13 in terms of the mean and standard deviation of the error values (*f*(*x*) − *f*(*∗*)) obtained in the 30 runs independently by EFLA with different parameter combinations, and the bold font denotes the winner. The character ‘R' in the first line of Table 13 is the abbreviation of word ‘rank'; each column starting with ‘R' after each EFLA algorithm means the rank of the different twelve parameter combinations. The last line of Table 13 shows the number of winners for the EFLA by different parameter combinations. In order to analyze the impact of population size (popsize) of EFLA, the twelve parameter combinations are arranged to six groups as popsize = 20 (EFLA01, EFLA02, EFLA03, and EFLA04), popsize = 30 (EFLA05), popsize = 40 (EFLA06), popsize = 50 (FELA07), popsize = 60 (EFLA08), and popsize = 100 (EFLA09, EFLA10, EFLA11, and EFLA12). Generally speaking, the performances of many metaheuristic algorithms are affected by the population size. The larger population size can enhance the diversity of population but can reduce the convergence speed. Therefore, the population size of EFLA like other algorithms should be tuned according to the different optimization problems. In Table 13, it can be observed that EFLAs (EFLA01, EFLA02, EFLA03, and EFLA04) by the minimal population size (popsize = 20) obtain the larger number of winners especially for the Type 1 (basic unrotated benchmark functions, F1–F15). Contrast to the Type 2 (F16–F30, the rotated, composition, and hybrid problems), EFLAs (from EFLA05 to EFLA12) corresponding to the population size (from popsize = 30 to popsize = 100) obtain the larger number of winners especially for the Type 2. It can be observed that EFLAs can obtain better performance for Type 1 and Type 2 problems when the population size is increased from 30 to 60. In addition, the other two parameter combinations (*m, n*) also affect the performance of EFLA by the same population size. According to equations (6) and (7), we know that the number of submemeplexes (*m*) is equal to the number of the best solution (*X*_*best*_), which influences the first potential well *P*_*k*_. EFLA with smaller number of submemeplexes is easy to trap into the local optimum for the multimodal problems due to the small numbers (parameter *m*) of the best solution (*X*_*best*_). In contrast, the larger number of submemeplexes (*m*) can increase the diversity of the population but cannot ensure that it obtains better solution.  Figure 6 shows the performance of EFLAs with different parameter combinations by Friedman's test. It can be observed that EFLA obtains the poor performance by the smaller values of *m* (*m* = 2 for population size 20 or 100) whether the population size is larger or smaller.  Table 14 shows the average rank results by the Friedman test. We can see that the best parameter combination of *popsize, m*, and *n* is (popsize = 50, *m* = 10, and *n* = 5).  Table 15 shows the statistical value (*p*−value = 0.003); it indicates that the performance of EFLA with different four parameters has significant difference. In addition, we compare the performance of the 12 algorithms with that of the EFLA algorithms with the 12 different parameter combinations by Friedman's test. The statistical value is equal to 200.829, and *p* value is equal to 2.40E−30. It means that there are significant differences among the 24 algorithms.  Figure 7 shows the ranks among the 24 algorithms. It is worth mentioning that the EFLA outperforms all the 12 algorithms no matter which parameter combination is chosen.

The article "An Evolutionary Frog Leaping Algorithm for Global Optimization Problems and Applications" was published in 2021. Journal: Comput Intell Neurosci.

### 5.4. The Time Complexity of EFLA Algorithm

#### 5.4.1. Theoretical Analysis for the Time Complexity

In this paper, the time complexity of the proposed method depends on the number of fitness evaluation, number of iterations, population size, covariance matrix, and eigen decomposition. So, the overall time complexity can be presented as follows:

(21) $$\begin{array}{c} O\left(\text{EFLA}\right)=O\left(QE\right)+O\left(AEE\right), \end{array}$$

where *QE* means the time complexity of quantum evolution (QE) operator and AEE means the time complexity of adaptive eigenvector evolution (AEE) operator. For the quantum evolutionary operator, the time complexity of the potential well is *O*(*n*), where *n* is the number of frogs in each submemeplex. Thus, the total time complexity of *QE* is as follows:

(22) $$\begin{array}{c} O\left(QE\right)=O\left(m*n*n*T*D\right)=O\left(ps*n*T*D\right), \end{array}$$

where *ps* is the population size, *m* is the number of submemeplexes, *n* is the number of frogs, *ps*=*m∗n*, *T* is the number of iteration, and *D* is the dimension. For the time complexity of the eigenvector evolutionary operator (EE), the covariance matrix contains *D∗D* elements, each of which requires *ps* cycles to be done. The eigen decomposition is solved by Jacobi's method, of which the time complexity is *O*(*D*^3^). In the proposed method, the adaptive evolutionary operator is completed. Thus, in extreme cases, if all the individuals in population achieve the eigenvector evolutionary operator, the overall time complexity of the eigenvector evolution is as follows:

(23) $$\begin{array}{c} O\left(EE\right)=O\left(D^{2}*ps*T\right)+O\left(D^{3}*T\right). \end{array}$$

In another case, if all the individuals in the population achieve the basic evolutionary operator (*BE*), the overall time complexity is as follows:

(24) $$\begin{array}{c} O\left(BE\right)=O\left(ps*T*D\right). \end{array}$$

So, *O*(*BE*) ≤ *O*(AEE) ≤ *O*(*EE*).

Therefore, in the worst case, the overall time complexity of EFLA is as follows:

(25) $$\begin{array}{c} O\left(\text{EFLA}\right)=O\left(ps*n*T*D\right)+O\left(D^{2}*ps*T\right)+O\left(D^{3}*T\right). \end{array}$$

In the best case, the overall time complexity of EFLA is as follows:

(26) $$\begin{array}{c} O\left(\text{EFLA}\right)=O\left(ps*n*T*D\right)+O\left(ps*T*D\right). \end{array}$$

#### 5.4.2. Experimental Results and Analysis for the Running times

All the algorithms are run by Matlab R2016a using the Windows 7 operating system. Hardware configuration of the computer is as follows: four CPU, Intel (R) Core (TM) i5−4200 U, CPU 1.60 GHz, and RAM 4.00 GB. Five optimization problems (F26, F27, F28, F29, and F30) in Table 1 are adopted. We select these five functions because they are hybrid functions or composition functions, which means that these problems are more complex and need more running times. Each algorithm is run 30 times for each optimization problem independently, and all the running times (minutes) are saved. All the parameter settings of the 13 algorithms are adopted as mentioned above. The experimental results are shown in Table 16. The character ‘**R**' in the first line of Table 16 is the abbreviation of word ‘rank'; each column starting with ‘**R**' after each algorithm denotes the rank of the 13 algorithms. The bold fonts denote the winner for the running times. In addition, the second column and the third column denote the rank and averages rank value by the Friedman test, where the *p* value = 3.14*E* − 4, and the statistical value = 36.0791. It can be observed that the rank of the 13 algorithms is GbABC (R_All = 1), LAPO (R_All = 2), AAA (R_All = 3), **EFLA (R_All** **=** **4)**, WQPSO (R_All = 5), SFLA (R_All = 6), SSA (TSQPSO) (R_All = 7), NNA (SCA) (R_All = 8), GWO (R_All = 9), CMAES (R_All = 10), and SaDE (R_All = 11). Although LAPO and GbABC obtain the better running time than other algorithms, they cannot obtain the better performance than many algorithms (it can be seen in Table 3**)**. The classical algorithms such as SaDE and CMAES obtain the worst running times although they can obtain the better performance for some problems. EFLA obtains the best performance than the other 12 algorithm (it can be seen in Table 3) by an acceptable running time.

The article "An Evolutionary Frog Leaping Algorithm for Global Optimization Problems and Applications" was published in 2021. Journal: Comput Intell Neurosci.

### 5.5. Experiment on the Parameter Optimization of SVM

Support vector machine (SVM) is a statistical classification method based on the VC (Vapnik–Chervonenkis) statistical learning theory and the structural risk minimization principle proposed by Vapnik et al. [77], which has been applied widely to many fields. Given a set of training data samples as {(*x*_1_, *y*_1_), (*x*_2_, *y*_2_),…, (*x*_*l*,_*y*_*l*_)} ∈ {(*x* × *y*)^*l*^}, *i*=1,2,…, *l*, where *x*_*i*_ ∈ *x* ⊂ *R*^*n*^ represents the input vector and *y*_*i*_={−1, +1} represents the number of class. The task of classification is to find the maximum margin separating hyper plane. It is an optimal problem, which can be represented as follows:

(27) $$\begin{array}{c} \min\;\frac{1}{2}\overset{l}{\underset{i,j=1}{\sum }}y_{i}y_{j}\alpha_{i}\alpha_{j}K\left(x_{i}\cdot x_{j}\right)-\overset{l}{\underset{j=1}{\sum }}\alpha_{j},\\ \text{s.t.}\;\overset{l}{\underset{i=1}{\sum }}y_{i}\alpha_{i}=0,\;\left(0\leq \alpha_{i}\leq C,i=1,2,\ldots ,l\right), \end{array}$$

where *K*(·, ·) denotes the kernel function, *K*(*x*_*i*_, *x*_*j*_)=exp(−‖*x*_*i*_ − *x*_*j*_‖^2^/2*σ*^2^) is the generally used kernel functions, and *σ* is a parameter. Experiments show that the parameters (*C*, *σ*) should be tuned before SVM is used. It can be seen as a black box optimization problem and can be solved by the metaheuristic algorithms.

The article "An Evolutionary Frog Leaping Algorithm for Global Optimization Problems and Applications" was published in 2021. Journal: Comput Intell Neurosci.

In this test, six benchmark data sets chosen from machine learning databases [78] are used for the LIBSVM tool provided by Chih-Jen Lin [79]. To achieve the parameter optimization, the searching space of (*C*, *σ*) is set as [1E−1, 1E3] for *C* and [1E−2, 1E3] for *σ*. The accuracy of prediction (%) of SVM by the 10-cross validation is used as the fitness value. For fair comparison, the parameter setting including the population size is set as Table 17 according to the related literature, and the max fitness evaluation is set as MAX_FES = 1000. Four methods including LSHADE [20], LSHADE-EpSin [65], TLBO [8], and LAPO [69] are selected for comparison. And the parameter settings of LSHADE and LSHADE-EpSin are used as literatures [20, 65]. Specifically, LSHADE obtains the winner in CEC 2014 and LSHADE-EpSin obtains the winner in CEC 2016. Each algorithm is run 20 times, and the median, mean, and std. are recorded for comparison.

Table 18 shows the details of the six data sets with different dimension.  Table 19 shows the median and std. of the five algorithms for six data sets. We can see that EFLA obtains the best accuracy of prediction than LSHADE, LSHADE-cnEpSin, TLBO, and LAPO for PBCW data set (F4) in high dimension and heart data set (F6) in low dimension space. It indicates the better scalability of EFLA to solve the parameter optimization problems of SVM. EFLA obtains the same accuracy of LSHADE, LSHADE-cnEpSin, TLBO, and LAPO for F2, F3, and F5.

In addition, we draw the convergence curve as Figure 8 for the fair comparison including the search speed and the accuracy. In the early iteration, the proposed algorithm does not converge faster than the other algorithms. It means that it has stronger exploration ability and is not easy to trap into the local optimum. In the late iteration, the proposed algorithm jumps out the local optimum and finds the better solution. To sum up, we can see that EFLA has better performance than LSHADE, LSHADE-cnEpSin, TLBO, and LAPO.

## 6. Conclusions

In this paper, we propose an improved SFLA algorithm (called EFLA) by the quantum evolutionary operator and the adaptive eigenvector evolutionary operator. The quantum evolutionary operator is used as the local search step instead of the traditional guidance mechanism, and the adaptive eigenvector evolutionary operator is used as the global search step instead of only using the shuffled operator. In addition, the basic search rule and the eigenvector search rule are chosen alternately to solve more different optimization problems in the coordinate system or in the rotated coordinate system. The adaptive eigenvector evolutionary operator enhances the search ability to solve the optimization problems in the rotated coordinate system.

The article "An Evolutionary Frog Leaping Algorithm for Global Optimization Problems and Applications" was published in 2021. Journal: Comput Intell Neurosci.

Then, we compare the proposed approach with the 15 well−known algorithms by the best parameter setting including NNA, SSA, SCA, SFLA, LAPO, CMAES, GWO, GbABC, WQPSO, TSQPSO, SaDE, AAA, TLBO, LSHADE, and LSHADE−cnEpSin for the 30 benchmark problems and real−world parameter optimization problems of SVM. The *T*-test, Wilcoxon signed-rank test, and Friedman's test are used to verify the performance of EFLA. In addition, we analyze the influence of the three major parameters of EFLA: popsize, *m*, and *n*. In general, we recommend that the three parameters (*popsize, m,* and *n*) can be set as [5, 6, 30] or [5, 10, 50] according to the experimental results and analysis. Finally, we analyze the time complexity of the EFLA algorithm and compare the running time of it with that of the 12 other algorithms. We obtain the accepted running time of EFLA with the best performance than the others (rank = 4).

In future, the proposed algorithm can be considered to solve more real-world continuous optimization problems in different fields. Such as, it may be used for an experimental evolutionary model in the domain of magnetorheological fluids [80]. Second, the quantum evolutionary operator can be used to improve the performance of the other heuristic algorithms. Third, the proposed eigenvector evolution method can be extended to solve other problems.

## Figures and Tables

**Figure 1:** Quantum evolutionary process.

**Figure 2:** Shifted rotated expanded Scaffers F6.

**Figure 3:** Adaptive eigenvector evolutionary operator.

**Figure 4:** Convergence curve: (a) F3 Schwefel's problem 1.2; (b) F7 Griewank function; (c) F11 Zakharov function; (d) F15 inverted cosine mixture problem; (e) F21 rotated Schwefel's function; (f) F25 hybrid function 2 (*N* = 3); (g) F26 hybrid function 4 (*N* = 4); (h) F27 hybrid function 5 (*N* = 5); (i) F28 hybrid function 6 (*N* = 5).

**Figure 5:** Convergence curve: (a) F23 rotated Schwefel's function; (b) F28 hybrid function 4(*n* = 4).

**Figure 6:** Comparison of parameter setting.

**Figure 7:** Comparison of parameter setting.

**Figure 8:** (a) Glass; (b) wine; (c) OBCW; (d) PBCW; (e) WDBC; (f) heart.

**Algorithm 1:** Pseudo code of SFLA.

**Algorithm 2:** Pseudo code.

**Table 1:** Details of benchmark problem.

Fun	Benchmark problem	Type low	Low	Up	Dim	Optimum values
F1	Sphere function	U	−100	100	30	0
F2	Schwefel's problem 2.22	U	−10	10	30	0
F3	Schwefel's problem 1.2	U	−100	100	30	0
F4	Quartic function	U	−1.28	1.28	30	0
F5	Rastrigrin function	M	−5.12	5.12	30	0
F6	Ackley function	M	−32	32	30	0
F7	Griewank function	M	−600	600	30	0
F8	Rosenbrock function	M	−10	10	30	0
F9	Penalized function	M	−50	50	30	0
F10	Weierstrass's function	M	−0.5	0.5	30	0
F11	Zakharov function	M	−5	10	30	0
F12	Alpine function	M	−10	10	30	0
F13	Salomon problem	M	−100	100	30	0
F14	Periodic problem	M	−10	10	30	0.9
F15	Inverted cosine mixture problem	M	−1	1	30	0
F16	Sphere function	U	−100	100	30	−1400
F17	Rotated high conditioned elliptic function	U	−100	100	30	−1300
F18	Rotated discus function	U	−100	100	30	−1100
F19	Different powers function	U	−100	100	30	−1000
F20	Rotated Ackley's function	M	−100	100	30	−700
F21	Rotated Weierstrass function	M	−100	100	30	−600
F22	Rotated Griewank's function	M	−100	100	30	−500
F23	Rotated Schwefel's function	M	−100	100	30	100
F24	Expanded Scaffer's F6 function	M	−100	100	30	600
F25	Shifted and rotated Schwefel's function	M	−100	100	30	1100
F26	Hybrid function 1 (N = 3)	M	−100	100	30	1700
F27	Hybrid function 2 (N = 3)	M	−100	100	30	1800
F28	Hybrid function 4 (N = 4)	M	−100	100	30	2000
F29	Hybrid function 5 (N = 5)	M	−100	100	30	2100
F30	Composition function 2 (N = 3)	M	−100	100	30	2400

The article "An Evolutionary Frog Leaping Algorithm for Global Optimization Problems and Applications" was published in 2021. Journal: Comput Intell Neurosci.

**Table 2:** Parameters setting.

No.	Algorithm	Parameter setting
1	NNA [68]	w = 1/(2 *∗* log(2)), c1 = 0.5 + log(2), c2 = c1, pop_size = 50
2	LAPO [69]	F = 0.5, CR = 0.9, pop_size = 40
3	GbABC [70]	SN = 12, limit = 1.12 *∗* (popsize/2) *∗* D, C = 1.507, pop_size = 24
4	SFLA [38]	c = 1, le = 5, m = 8, n = 5, pop_size = 40
5	SCA [72]	pmodify = 1, PMutate = 0.01, elitism parameter = 2, pop_size = 30
6	SSA [11]	Rpower = 2, Rnorm = 2, ElitistCheck = 1, pop_size = 30
7	GWO [6]	pop_size = 30
8	CMAES [73]	*σ*=0.25, *μ*=floor(4+floor(3 · log(*D*))/2) pop_size = 4 + floor(3 log (D)), D is the dimension
9	WQPSO [48]	W = Wmin + (MAX_FES-FES)/MAX_FES *∗* (Wmax-Wmin), Wwin = 0.5, Wmax = 1.0, pop_size = 80
10	TSQPSO [57]	W = Wmin + (MAX_FES-FES)/MAX_FES *∗* (Wmax−Wmin), Wwin = 0.5, Wmax = 1.0, pop_size = 50
11	SaDE [74]	F ∼N (0.5, 0.3), CR ∼N (CRm, 0.1), mutation strategies and crossover strategies, learngen = 50; pop_size = 50
12	AAA [10]	e = 0.3, delta = 2, Ap = 0.5, pop_size = 40
13	EFLA	m = 6, n = 5, pop_size = 30

**Table 3:** Comparison results of EFLA and other algorithms.

Func	LAPO	**R**	TSQPSO	**R**	WQPSO	**R**	GbABC	**R**	NNA	**R**	SaDE	**R**	EFLA	**R**
F1 mean	2.0679*E* − 148	**4**	2.6238*E* − 211	**3**	4.8770*E* − 113	**6**	2.9012*E* − 16	**12**	2.7095*E* − 17	**11**	9.1574*E* − 131	**5**	**1.9097** *E* − **232**	**1**
Std.	4.2386*E* − 148		0.0000*E* + 00		1.7583*E* − 112		5.0880*E* − 17		4.6804*E* − 17		3.4926*E* − 130		**0.0000*E*** + **00**	
F2 mean	3.7638*E* − 149	**4**	7.8721*E* − 211	**3**	4.2486*E* − 114	**6**	2.7007*E* − 16	**12**	1.6208*E* − 19	**11**	1.0352*E* − 131	**5**	3.3520*E* − 233	**2**
Std.	1.8902*E* − 148		0.0000*E* + 00		1.1122*E* − 113		4.5535*E* − 17		2.6731*E* − 19		4.1658*E* − 131		0.0000*E* + 00	
F3 mean	3.6017*E* − 33	**2**	4.1406*E* − 03	**8**	4.2179*E* − 01	**9**	1.7557*E* + 03	**13**	1.6058*E* − 09	**6**	5.2152*E* − 07	**7**	**3.3911*E* − 34**	**1**
Std.	1.9395*E* − 32		7.0602*E* − 03		1.3847*E* + 00		1.1055*E* + 03		3.5930*E* − 09		1.1523*E* − 06		**1.5866*E* − 33**	
F4 mean	**4.7463*E* − 05**	**1**	3.7149*E* − 04	**4**	1.1896*E* − 03	**5**	2.2604*E* − 02	**12**	2.6980*E* − 04	**3**	2.5599*E* − 03	**8**	1.7149*E* − 03	**6**
Std.	**3.2024*E* − 05**		1.6593*E* − 04		3.9106*E* − 04		5.1604*E* − 03		1.5368*E* − 04		1.0640*E* − 03		1.0814*E* − 03	
F5 mean	**0.0000*E*** + **00**	**1**	1.0518*E* + 02	**9**	1.5472*E* + 01	**5**	**0.0000*E*** + **00**	**1**	4.0321*E* + 01	**7**	**0.0000*E*** + **00**	**1**	**0.0000*E*** + **00**	**1**
Std.	**0.0000*E*** + **00**		2.9610*E* + 01		3.6786*E* + 00		**0.0000*E*** + **00**		3.2685*E* + 01		**0.0000*E*** + **00**		**0.0000*E*** + **00**	
F6 mean	1.0463*E* + 01	**9**	**4.5001*E* − 15**	**1**	5.6843*E* − 15	**2**	2.9132*E* − 14	**5**	8.2543*E* − 10	**6**	6.2087*E* − 02	**7**	7.2239*E* − 15	**3**
Std.	8.3330*E* − 01		**1.5979*E* − 15**		1.7702*E* − 15		2.3603*E* − 15		1.2301*E* − 09		2.3628*E* − 01		1.4703*E* − 15	
F7 mean	1.8553*E* − 03	**5**	3.6281*E* − 04	**3**	9.8442*E* − 03	**8**	**0.0000*E*** + **00**	**1**	1.9066*E* − 03	**6**	4.5956*E* − 03	**7**	**0.0000*E*** + **00**	**1**
Std.	1.0162*E* − 02		1.9827*E* − 03		1.1601*E* − 02		**0.0000*E* + 00**		7.4693*E* − 03		8.9739*E* − 03		**0.0000*E*** + **00**	
F8 mean	2.8902*E* + 01	**11**	2.5087*E* + 01	**7**	2.4225*E* + 01	**6**	2.6748*E* + 00	2	2.5286*E* + 01	**8**	2.3092*E* + 01	**5**	1.9977*E* + 01	**4**
Std.	3.0136*E* − 02		1.6761*E* − 01		1.0980*E* + 01		1.2591*E* + 01		1.0413*E* + 01		9.8351*E* + 00		7.8322*E* − 01	
F9 mean	5.8221*E* − 01	**10**	9.4438*E* − 06	**5**	1.5715*E* − 06	**3**	2.5623*E* − 16	**2**	7.3370*E* − 06	**4**	3.4556*E* − 03	**6**	4.4920*E* − 02	**9**
Std.	1.2562*E* − 01		7.7667*E* − 06		2.0857*E* − 07		3.1052*E* − 17		1.1419*E* − 05		1.8927*E* − 02		1.1119*E* − 01	
F10 mean	**0.0000*E*** + **00**	**1**	**0.0000*E*** + **00**	**1**	**0.0000*E*** + **00**	**1**	**0.0000*E*** + **00**	**1**	1.4559*E* − 07	**2**	4.8788*E* − 03	**3**	**0.0000*E*** + **00**	**1**
Std.	**0.0000*E*** + **00**		**0.0000*E*** + **00**		**0.0000*E*** + **00**		**0.0000*E*** + **00**		2.9588*E* − 07		2.1574*E* − 02		**0.0000*E*** + **00**	
F11 mean	7.0369*E* − 57	**2**	6.0621*E* − 24	**6**	3.1426*E* − 15	**8**	1.5685*E* + 02	**13**	3.3002*E* − 16	**7**	1.4262*E* − 12	**9**	**4.0066*E* − 75**	**1**
Std.	2.5996*E* − 56		2.4055*E* − 23		3.7257*E* − 15		4.1783*E* + 01		4.9773*E* − 16		2.7601*E* − 12		**1.6367*E* − 74**	
F12 mean	3.4937*E* − 81	**2**	3.8208*E* − 01	**11**	6.7492*E* − 03	**9**	8.5518*E* − 08	**7**	3.5388*E* + 00	**13**	2.0354*E* − 17	**4**	4.9165*E* − 16	**6**
Std.	5.3073*E* − 81		2.0428*E* + 00		1.3164*E* − 02		4.6840*E* − 07		2.2808*E* + 00		1.1148*E* − 16		8.0839*E* − 16	
F13 mean	**9.9873*E* − 02**	**1**	1.6654*E* − 01	**5**	2.0321*E* − 01	**7**	6.5987*E* − 01	**12**	1.5321*E* − 01	**4**	2.5654*E* − 01	**8**	1.9987*E* − 01	**6**
Std.	**2.6587*E* − 09**		4.7946*E* − 02		3.1984*E* − 02		1.3287*E* − 01		5.0742*E* − 02		6.2606*E* − 02		2.6261*E* − 02	
F14 mean	2.2111*E* + 00	**11**	2.9183*E* + 00	**12**	1.2187*E* + 00	**10**	1.0000*E* − 01	**4**	1.4937*E* − 01	**6**	1.1274*E* − 01	**5**	1.6718*E* − 01	**7**
Std.	1.3244*E* + 00		7.6066*E* − 01		1.2750*E* + 00		1.8426*E* − 06		7.6006*E* − 02		5.4024*E* − 03		4.8375*E* − 02	
F15 mean	6.1931*E* − 151	**4**	1.7370*E* − 214		2.4477*E* − 116	**5**	5.1648*E* − 17	**9**	1.3067*E* − 20	**8**	4.9261*E* − 03	**11**	2.3950*E* − 236	**2**
Std.	1.9234*E* − 150		0.0000*E* + 00		1.0387*E* − 115		6.3433*E* − 18		3.9609*E* − 20		2.6982*E* − 02		0.0000*E* + 00	
F16 mean	4.9333*E* + 04	**13**	3.4645*E* + 00	**9**	3.2837*E* − 01	**7**	6.2149*E* − 13	**6**	2.2862*E* + 00	**8**	**0.0000*E*** + **00**	**1**	3.7138*E* − 13	**4**
Std.	3.4293*E* + 03		7.6157*E* + 00		4.6514*E* − 02		1.4545*E* − 13		4.0603*E* + 00		**0.0000*E*** + **00**		1.9333*E* − 13	
F17 mean	6.2032*E* + 08	**13**	7.2635*E* + 06	**7**	4.4582*E* + 06	**6**	1.7429*E* + 07	**9**	1.2600*E* + 07	**8**	4.2644*E* + 05	**3**	1.5593*E* + 05	**2**
Std.	2.4118*E* + 08		2.8245*E* + 06		2.2790*E* + 06		5.2228*E* + 06		4.3819*E* + 06		2.4265*E* + 05		1.0031*E* + 05	
F18 mean	6.4263*E* + 04	**12**	1.4323*E* + 03	**3**	2.1750*E* + 03	**4**	8.7421*E* + 04	**13**	9.6899*E* + 03	**8**	3.1923*E* + 03	**6**	5.5248*E* + 00	**2**
Std.	3.1371*E* + 03		6.4265*E* + 02		9.1906*E* + 02		1.2549*E* + 04		3.9949*E* + 03		1.5177*E* + 03		5.3507*E* + 00	
F19 mean	1.9648*E* + 04	**13**	4.4660*E* + 01	**10**	2.3662*E* − 01	**7**	1.1823*E* − 12	**4**	1.5171*E* + 00	**8**	**0.0000*E*** + **00**	**1**	6.0633*E* − 13	**3**
Std.	6.7840*E* + 03		1.5296*E* + 01		2.6707*E* − 02		2.9945*E* − 13		2.9757*E* + 00		**0.0000*E*** + **00**		3.3022*E* − 13	
F20 mean	2.0942*E* + 01	**8**	2.0945*E* + 01	**9**	2.0936*E* + 01	**5**	2.0957*E* + 01	**12**	2.0952*E* + 01	**10**	2.0930*E* + 01	**3**	2.0921*E* + 01	**2**
Std.	6.6635*E* − 02		4.2900*E* − 02		4.8137*E* − 02		4.3188*E* − 02		4.7127*E* − 02		5.4512*E* − 02		6.9368*E* − 02	
F21 mean	3.3880*E* + 01	**12**	3.2223*E* + 01	**10**	1.9235*E* + 01	**2**	2.9199*E* + 01	**6**	2.9536*E* + 01	**8**	**1.7362*E*** + **01**	**1**	2.1746*E* + 01	**3**
Std.	1.1392*E* + 00		3.2294*E* + 00		3.9092*E* + 00		2.2216*E* + 00		2.9798*E* + 00		**2.8439*E*** + **00**		3.2228*E* + 00	
F22 mean	7.5833*E* + 03	**13**	1.5974*E* + 01	**9**	1.3157*E* + 00	**7**	1.2354*E* + 00	**6**	9.9663*E* + 00	**8**	2.5310*E* − 01	**4**	2.1249*E* − 01	**3**
Std.	1.4622*E* + 03		1.1760*E* + 01		2.1498*E* − 01		4.0112*E* − 01		8.0468*E* + 00		1.2585*E* − 01		1.1696*E* − 01	
F23 mean	7.2429*E* + 03	**12**	5.9708*E* + 03	**9**	7.1367*E* + 03	**11**	3.9898*E* + 03	**3**	4.6973*E* + 03	**7**	4.5802*E* + 03	**6**	**3.0790*E*** + **03**	**1**
Std.	3.3604*E* + 02		9.0511*E* + 02		3.6869*E* + 02		4.3627*E* + 02		7.2290*E* + 02		1.1312*E* + 03		**5.8848*E*** + **02**	
F24 mean	1.2784*E* + 01	**9**	1.1985*E* + 01	**5**	1.1978*E* + 01	**4**	1.4554*E* + 01	**13**	1.2935*E* + 01	**11**	**1.0801*E*** + **01**	**1**	1.1167*E* + 01	**2**
Std.	3.8517*E* − 01		4.8984*E* − 01		4.4676*E* − 01		2.1412*E* − 01		7.5276*E* − 01		**5.1674*E* − 01**		8.5698*E* − 01	
F25 mean	6.6897*E* + 03	**10**	5.4734*E* + 03	**9**	5.3861*E* + 03	**12**	**2.0737*E*** + **03**	**1**	3.9468*E* + 03	**7**	3.1024*E* + 03	**4**	2.7380*E* + 03	**3**
Std.	3.2043*E* + 02		7.7868*E* + 02		1.2302*E* + 03		**3.5805*E*** + **02**		6.6736*E* + 02		6.7238*E* + 02		5.7139*E* + 02	
F26 mean	5.3508*E* + 07	**13**	2.1023*E* + 05	**4**	2.9649*E* + 05	**6**	5.9358*E* + 06	**11**	8.9966*E* + 05	**8**	1.0982*E* + 04	**3**	**9.3688*E*** + **02**	**1**
Std.	3.4832*E* + 07		1.2160*E* + 05		1.8309*E* + 05		3.7139*E* + 06		7.6690*E* + 05		1.1758*E* + 04		**2.7344*E*** + **02**	
F27 mean	3.8211*E* + 09	**13**	1.8409*E* + 03	**6**	7.7833*E* + 03	**8**	5.6953*E* + 04	**10**	2.6359*E* + 04	**9**	8.1686*E* + 02	**4**	**8.4483*E*** + **01**	**1**
Std.	1.5410*E* + 09		2.0800*E* + 03		7.8001*E* + 03		7.4420*E* + 04		4.8954*E* + 04		9.0611*E* + 02		**2.1385*E*** + **01**	
F28 mean	9.4589*E* + 04	**13**	2.8808*E* + 02	**4**	4.5894*E* + 02	**5**	1.0856*E* + 04	**11**	6.1975*E* + 03	**9**	**7.8279*E*** + **01**	**1**	8.5297*E* + 01	**2**
Std.	3.6264*E* + 04		1.8178*E* + 02		1.8715*E* + 02		4.4541*E* + 03		4.2717*E* + 03		**5.6083*E*** + **01**		4.1632*E* + 01	
F29 mean	1.1208*E* + 07	**13**	8.1877*E* + 04	**5**	8.0641*E* + 04	**4**	8.2012*E* + 05	**11**	3.6377*E* + 05	**9**	3.8309*E* + 03	**3**	**4.1560*E*** + **02**	**1**
Std.	9.9516*E* + 06		6.1105*E* + 04		7.9208*E* + 04		4.8406*E* + 05		2.8624*E* + 05		3.7988*E* + 03		**1.6027*E*** + **02**	
F30 mean	**2.0000*E*** + **02**	**1**	2.1146*E* + 02	**4**	2.2985*E* + 02	**11**	2.2947*E* + 02	**10**	2.2436*E* + 02	**6**	2.2694*E* + 02	**9**	2.1221*E* + 02	**5**
Std.	**2.0568** *E* − **03**		1.4433*E* + 01		6.0633*E* + 00		1.1562*E* + 00		1.4539*E* + 01		4.0580*E* + 00		1.3611*E* + 01	

The article "An Evolutionary Frog Leaping Algorithm for Global Optimization Problems and Applications" was published in 2021. Journal: Comput Intell Neurosci.

**Table 4:** Comparison results of EFLA and other algorithms.

Func	SFLA	**R**	SSA	**R**	CMAES	**R**	SCA	**R**	AAA	**R**	GWO	**R**	EFLA	**R**
F1 mean	1.4983*E* − 14	**13**	1.8953*E* − 52	**8**	1.8594*E* − 29	**10**	3.0185*E* − 52	**9**	7.7636*E* − 81	**7**	3.9830*E* − 229	**2**	**1.9097*E* − 232**	**1**
Std.	6.8321*E* − 14		3.0968*E* − 53		2.1514*E* − 30		1.4485*E* − 51		1.1026*E* − 80		0.0000*E* + 00		**0.0000*E*** + **00**	
F2 mean.	4.1071*E* − 16	**13**	1.8339*E* − 54	**8**	1.9386*E* − 29	**10**	8.0787*E* − 52	**9**	1.0913*E* − 83	**7**	**7.7509*E* − 234**	**1**	3.3520*E* − 233	**2**
Std.	2.1422*E* − 15		3.7522*E* − 55		2.1448*E* − 30		4.4249*E* − 51		1.8890*E* − 83		**0.0000*E*** + **00**		0.0000*E* + 00	
F3 mean	1.0252*E* + 01	**11**	7.5471*E* − 11	**5**	7.0456*E* − 28	**3**	2.0687*E* + 01	**12**	6.0855*E* + 00	**10**	9.8559*E* − 27	**4**	**3.3911*E* − 34**	**1**
Std.	4.6762*E* + 00		1.5092*E* − 10		9.4987*E* − 29		1.0603*E* + 02		4.4564*E* + 00		4.0907*E* − 26		**1.5866*E* − 33**	
F4 mean	2.0006*E* − 03	**7**	1.7915*E* − 02	**11**	5.5304*E* − 02	**13**	2.6205*E* − 03	**9**	9.4294*E* − 03	**10**	2.2596*E* − 04	**2**	1.7149*E* − 03	**6**
Std.	5.2913*E* − 04		6.7959*E* − 03		1.5263*E* − 02		2.6535*E* − 03		2.2864*E* − 03		1.1757*E* − 04		1.0814*E* − 03	
F5 mean	1.9710*E* + 01	**6**	6.6961*E* + 01	**8**	2.3242*E* + 02	**10**	1.2529*E* + 00	**4**	3.3165*E* − 02	**2**	8.2594*E* − 01	**3**	**0.0000*E*** + **00**	**1**
Std.	7.1148*E* + 00		1.3697*E* + 01		4.9397*E* + 01		6.8622*E* + 00		1.8165*E* − 01		2.0051*E* + 00		**0.0000*E*** + **00**	
F6 mean	2.0516*E* − 01	**8**	1.8791*E* + 00	**10**	1.9416*E* + 01	**13**	6.0329*E* + 00	**11**	1.3145*E* − 14	**4**	1.0121*E* + 01	**12**	7.2239*E* − 15	**3**
Std.	3.8173*E* − 01		9.6749*E* − 01		2.0146*E* − 01		9.3730*E* + 00		2.1173*E* − 15		1.0294*E* + 01		1.4703*E* − 15	
F7 mean	3.8681*E* − 02	**10**	1.0916*E* − 02	**9**	1.5606*E* − 03	**4**	**0.0000*E*** + **00**	**1**	**0.0000*E*** + **00**	**1**	2.7034*E* − 04	**2**	**0.0000*E*** + **00**	**1**
Std.	2.9514*E* − 02		1.0414*E* − 02		3.7436*E* − 03		**0.0000*E*** + **00**		**0.0000*E*** + **00**		1.4807*E* − 03		**0.0000*E*** + **00**	
F8 mean	3.0799*E* + 01	**12**	3.4417*E* + 01	**13**	**2.6577*E* − 01**	**1**	2.7378*E* + 01	**10**	8.4609*E* + 00	**3**	2.5979*E* + 01	**9**	1.9977*E* + 01	**4**
Std.	1.3159*E* + 01		2.3269*E* + 01		**1.0114*E*** + **00**		6.8511*E* − 01		1.4282*E* + 01		5.3992*E* − 01		7.8322*E* − 01	
F9 mean	3.4562*E* − 03	**6**	2.4483*E* + 00	**12**	6.9113*E* − 03	**7**	3.5419*E* − 01	**11**	**1.5705*E* − 32**	**1**	7.9047*E* − 03	**8**	4.4920*E* − 02	**9**
Std.	1.8927*E* − 02		2.2790*E* + 00		2.6302*E* − 02		8.5982*E* − 02		**5.5674*E* − 48**		7.8180*E* − 03		1.1119*E* − 01	
F10 mean	2.3550*E* + 00	**4**	1.3917*E* + 01	**6**	2.7419*E* + 00	**5**	**0.0000*E*** + **00**	**1**	**0.0000*E*** + **00**	**1**	**0.0000*E*** + **00**	**1**	**0.0000*E*** + **00**	**1**
Std.	1.0955*E* + 00		3.3271*E* + 00		2.0527*E* + 00		**0.0000*E*** + **00**		**0.0000*E*** + **00**		**0.0000*E*** + **00**		**0.0000*E*** + **00**	
F11 mean	4.0243*E* + 00	**12**	3.1346*E* − 45	**4**	2.9481*E* − 27	**5**	2.5242*E* − 07	**10**	1.3122*E* − 01	**11**	2.7033*E* − 45	**3**	**4.0066*E* − 75**	**1**
Std.	1.9618*E* + 00		1.7163*E* − 44		3.8367*E* − 28		5.3396*E* − 07		1.5176*E* − 01		8.5571*E* − 45		**1.6367*E* − 74**	
F12 mean	1.8256*E* − 04	**8**	2.7640*E* + 00	**12**	9.1571*E* − 02	**10**	8.8684*E* − 35	**3**	3.7515*E* − 16	**5**	**4.0050*E* − 142**	**1**	4.9165*E* − 16	**6**
Std.	5.1853*E* − 04		1.3874*E* + 00		1.4377*E* − 01		4.8574*E* − 34		7.4335*E* − 16		**2.1936*E* − 141**		8.0839*E* − 16	
F13 mean	4.1654*E* − 01	**10**	5.3321*E* − 01	**11**	2.8746*E* + 01	**13**	**1.0987*E* − 01**	**2**	4.1331*E* − 01	**9**	1.4987*E* − 01	**3**	1.9987*E* − 01	**6**
Std.	5.9209*E* − 02		8.4418*E* − 02		9.6013*E* + 00		**3.0513*E* − 02**		6.8037*E* − 02		5.0855*E* − 02		2.6261*E* − 02	
F14 mean	1.8365*E* − 01	**8**	1.0000*E* − 01	**2**	1.0000*E* − 01	**1**	1.5591*E* + 00	**9**	1.0000*E* − 01	**3**	5.9277*E* + 00	**13**	1.6718*E* − 01	**7**
Std.	2.2196*E* − 01		1.0506*E* − 16		7.0575*E* − 17		1.7118*E* + 00		1.0811*E* − 16		3.7705*E* − 01		4.8375*E* − 02	
F15 mean	3.3461*E* − 04	**10**	1.2266*E* + 00	**13**	3.1035*E* − 01	**12**	9.7236*E* − 54	**7**	1.2226*E* − 84	**6**	**5.3910*E* − 237**	**1**	2.3950*E* − 236	**2**
Std.	1.8095*E* − 03		4.0361*E* − 01		2.2413*E* − 01		5.3258*E* − 53		1.7662*E* − 84		**0.0000*E*** + **00**		0.0000*E* + 00	
F16 mean	1.9029*E* + 02	**10**	4.0927*E* − 13	**5**	3.0316*E* − 14	**2**	1.1694*E* + 04	**12**	2.6527*E* − 13	**3**	6.5110*E* + 02	**11**	3.7138*E* − 13	**4**
Std.	6.7655*E* + 01		1.3876*E* − 13		7.8614*E* − 14		1.5834*E* + 03		8.6186*E* − 14		4.5105*E* + 02		1.9333*E* − 13	
F17 mean	1.8713*E* + 07	**10**	3.5035*E* + 06	**5**	**2.2737*E* − 14**	**1**	1.3770*E* + 08	**12**	3.3818*E* + 06	**4**	1.9410*E* + 07	**11**	1.5593*E* + 05	**2**
Std.	2.9155*E* + 06		1.7388*E* + 06		**6.9378*E* − 14**		4.3839*E* + 07		2.3501*E* + 06		8.8776*E* + 06		1.0031*E* + 05	
F18 mean	1.0201*E* + 04	**9**	4.1146*E* + 03	**7**	**4.5475*E* − 14**	**1**	3.5670*E* + 04	**10**	3.7660*E* + 04	**11**	3.1308*E* + 03	**5**	5.5248*E* + 00	**2**
Std.	1.2569*E* + 03		2.1389*E* + 03		**9.2504*E* − 14**		5.3129*E* + 03		9.1768*E* + 03		1.6376*E* + 03		5.3507*E* + + 00	
F19 mean	8.5316*E* + 01	**9**	3.2161*E* − 03	**6**	2.4481*E* − 12	**5**	2.4590*E* + 03	**12**	2.6527*E* − 13	**2**	3.6569*E* + 02	**11**	6.0633*E* − 13	**3**
Std.	1.5073*E* + 01		2.9560*E* − 04		5.2136*E* − 12		8.6868*E* + 02		6.2149*E* − 14		2.0308*E* + 02		3.3022*E* − 13	
F20 mean	2.0960*E* + 01	**13**	**2.0908*E*** + **01**	**1**	2.0954*E* + 01	**11**	2.0939*E* + 01	**6**	2.0931*E* + 01	**4**	2.0941*E* + 01	**7**	2.0921*E* + 01	**2**
Std.	3.8597*E* − 02		**7.3270*E* − 02**		4.0485*E* − 02		5.7432*E* − 02		5.7590*E* − 02		5.4833*E* − 02		6.9368*E* − 02	
F21 mean	3.2559*E* + 01	**7**	2.6683*E* + 01	**5**	4.5021*E* + 01	**13**	3.9251*E* + 01	**11**	2.4122*E* + 01	**4**	3.3938*E* + 01	**9**	2.1746*E* + 01	**3**
Std.	3.1236*E* + 00		3.0815*E* + 00		6.6350*E* + 00		1.3787*E* + 00		2.4257*E* + 00		8.0021*E* + 00		3.2228*E* + 00	
F22 mean	6.6800*E* + 01	**10**	1.0450*E* − 01	**2**	**1.6916*E* − 02**	**1**	1.5845*E* + 03	**12**	2.3036*E* − 01	**5**	2.0064*E* + 02	**11**	2.1249*E* − 01	**3**
Std.	1.1481*E* + 01		4.5148*E* − 02		**1.1343*E* − 02**		3.5064*E* + 02		8.9844*E* − 02		1.0603*E* + 02		1.1696*E* − 01	
F23 mean	4.0343*E* + 03	**4**	4.2009*E* + 03	**5**	5.0284*E* + 03	**8**	7.4363*E* + 03	**13**	3.6318*E* + 03	**2**	7.0628*E* + 03	**10**	**3.0790*E*** + **03**	**1**
Std.	6.0325*E* + 02		6.7592*E* + 02		7.0278*E* + 02		2.3183*E* + 02		5.1933*E* + 02		6.7585*E* + 02		**5.8848*E*** + **02**	
F24 mean	1.2788*E* + 01	**10**	1.2548*E* + 01	**8**	1.2319*E* + 01	**6**	1.4018*E* + 01	**12**	1.2545*E* + 01	**7**	1.1801*E* + 01	**3**	1.1167*E* + 01	**2**
Std.	8.7092*E* − 01		1.2020*E* + 00		7.4841*E* − 01		3.1337*E* − 01		8.3427*E* − 01		5.8045*E* − 01		8.5698*E* − 01	
F25 mean	3.4020*E* + 03	**5**	3.8534*E* + 03	**6**	5.0874*E* + 03	**8**	6.9619*E* + 03	**11**	2.0730*E* + 03	**2**	5.8655*E* + 03	**13**	2.7380*E* + 03	**3**
Std.	7.3450*E* + 02		5.9094*E* + 02		6.8133*E* + 02		3.2297*E* + 02		4.3520*E* + 02		1.6214*E* + 03		5.7139*E* + 02	
F26 mean	1.3462*E* + 06	**9**	2.9059*E* + 05	**5**	1.5367*E* + 03	**2**	5.9984*E* + 06	**12**	7.7577*E* + 05	**7**	1.5977*E* + 06	**10**	**9.3688*E*** + **02**	**1**
Std.	3.6288*E* + 05		2.1346*E* + 05		3.6940*E* + 02		2.5093*E* + 06		5.0958*E* + 05		1.0360*E* + 06		**2.7344*E*** + **02**	
F27 mean	5.0549*E* + 02	**3**	5.4088*E* + 03	**7**	1.3463*E* + 02	**2**	1.4413*E* + 08	**12**	1.4795*E* + 03	**5**	2.5011*E* + 06	**11**	**8.4483*E*** + **01**	**1**
Std.	3.0414*E* + 02		5.9412*E* + 03		5.2506*E* + 01		8.8005*E* + 07		1.8325*E* + 03		6.0566*E* + 06		**2.1385*E*** + **01**	
F28 mean	5.3673*E* + 03	**8**	1.4662*E* + 03	**7**	3.0114*E* + 02	**3**	1.4684*E* + 04	**12**	7.2467*E* + 03	**10**	9.0622*E* + 02	**6**	8.5297*E* + 01	**2**
Std.	2.0421*E* + 03		1.3799*E* + 03		1.3330*E* + 02		5.6078*E* + 03		5.3916*E* + 03		1.4077*E* + 03		4.1632*E* + 01	
F29 mean	2.6622*E* + 05	**8**	1.0791*E* + 05	**6**	1.0405*E* + 03	**2**	1.4249*E* + 06	**12**	1.5329*E* + 05	**7**	4.9044*E* + 05	**10**	**4.1560*E*** + **02**	**1**
Std.	1.5496*E* + 05		8.1334*E* + 04		4.0995*E* + 02		4.6378*E* + 05		1.1548*E* + 05		4.5133*E* + 05		**1.6027*E*** + **02**	
F30 mean	2.2546*E* + 02	**8**	2.4364*E* + 02	**13**	2.3203*E* + 02	**12**	2.0010*E* + 02	**3**	2.2520*E* + 02	**7**	2.0001*E* + 02	**2**	2.1221*E* + 02	**5**
Std.	2.2867*E* + 00		5.6068*E* + 00		6.5750*E* + 00		9.8715*E* − 02		8.5013*E* − 01		3.8083*E* − 03		1.3611*E* + 01	

The article "An Evolutionary Frog Leaping Algorithm for Global Optimization Problems and Applications" was published in 2021. Journal: Comput Intell Neurosci.

**Table 5:** *T*-test for comparison results with EFLA and other algorithms.

Func	LAPO	TSQPSO	WQPSO	GbABC	NNA	SaDE
F1 *p* value	**6.1172*E* − 03**	0.0000*E* + 00	6.9769*E* − 02	**3.5402*E* − 24**	**1.7874*E* − 03**	8.0836*E* − 02
*t*-value	**2.6722*E*** + **00**	6.5535*E* + 04	1.5192*E* + 00	**3.1231*E*** + **01**	**3.1708*E*** + **00**	1.4361*E* + 00
F2 *p* value	1.4221*E* − 01	0.0000*E* + 00	**2.2638*E* − 02**	**1.1654*E* − 24**	**1.2156*E* − 03**	9.1988*E* − 02
*t*-value	1.0906*E* + 00	6.5535*E* + 04	**2.0923*E*** + **00**	**3.2486*E*** + **01**	**3.3210*E*** + **00**	1.3611*E* + 00
F3 *p* value	1.8380*E* − 01	**1.6081*E* − 03**	5.3001*E* − 02	**7.0531*E* − 10**	**1.0328*E* − 02**	**9.6192*E* − 03**
*t*-value	9.1528*E* − 01	**3.2122*E*** + **00**	1.6684*E* + 00	**8.6990*E*** + **00**	**2.4479*E*** + **00**	**2.4789*E*** + **00**
F4 *p* value	1.0000*E* + 00	1.0000*E* + 00	9.9181*E* − 01	**4.0816*E* − 20**	1.0000*E* + 00	**2.8020*E* − 03**
*t*-value	−8.4184*E* + 00	−6.7403*E* + 00	−2.5485*E* + 00	**2.2326*E*** + **0**1	−7.2306*E* + 00	**2.9924*E*** + **00**
F5 *p* value	**—**	**1.7304*E* − 18**	**1.7242*E* − 20**	**—**	**1.0224*E* − 07**	**—**
*t*-value	**—**	**1.9456*E*** + **01**	**2.3036*E*** + **01**	**—**	**6.7569*E*** + **00**	**—**
F6 *p* value	**5.6081*E* − 34**	1.0000*E* + 00	9.9988*E* − 01	**1.4270*E* − 29**	**4.7918*E* − 04**	8.0394*E* − 02
*t*-value	**6.8771*E*** + **01**	−8.3316*E* + 00	−4.1763*E* + 00	**4.8325*E*** + **01**	**3.6754*E*** + **00**	1.4392*E* + 00
F7 *p* value	1.6279*E* − 01	1.6225*E* − 01	**3.3740*E* − 05**	**—**	8.6346*E* − 02	**4.4460*E* − 03**
*t*-value	1.0000*E* + 00	1.0023*E* + 00	**4.6476*E*** + **00**	**—**	1.3981*E* + 00	**2.8049*E*** + **00**
F8 *p* value	**7.3722*E* − 33**	**1.0287*E* − 25**	**2.0964*E* − 02**	1.0000*E* + 00	**5.2738*E* − 03**	**4.4960*E* − 02**
*t*-value	**6.2889*E*** + **01**	**3.5394*E*** + **01**	**2.1284*E*** + **00**	−7.4374*E* + 00	**2.7342*E*** + **00**	**1.7544*E*** + **00**
F9 *p* value	**4.1085*E* − 17**	9.8251*E* − 01	9.8253*E* − 01	9.8253*E* − 01	9.8251*E* − 01	9.7187*E* − 01
*t*-value	**1.7285*E*** + **01**	−2.2123*E* + 00	−2.2127*E* + 00	−2.2127*E* + 00	−2.2124*E* + 00	−1.9886*E* + 00
F10 *p* value	**—**	**—**	**—**	**—**	**5.7935*E* − 03**	1.1271*E* − 01
*t*-value	**—**	**—**	**—**	**—**	**2.6950*E*** + **00**	1.2386*E* + 00
F11 *p* value	7.4481*E* − 02	8.9015*E* − 02	**3.6433*E* − 05**	**3.8744*E* − 19**	**5.3836*E* − 04**	**4.1812*E* − 03**
*t*-value	1.4826*E* + 00	1.3803*E* + 00	**4.6199*E*** + **00**	**2.0561*E*** + **01**	**3.6316*E*** + **00**	**2.8301*E*** + **00**
F12 *p* value	9.9882*E* − 01	1.5705*E* − 01	**4.4113*E* − 03**	1.6279*E* − 01	**1.1539*E* − 09**	9.9794*E* − 01
*t*-value	−3.3312*E* + 00	1.0244*E* + 00	**2.8081*E*** + **00**	1.0000*E* + 00	**8.4983*E*** + **00**	−3.1153*E* + 00
F13 *p* value	1.0000*E* + 00	9.9732*E* − 01	3.3119*E* − 01	**1.5281*E* − 17**	9.9983*E* − 01	**4.1641*E* − 05**
*t*-value	−2.0857*E* + 01	−3.0104*E* + 00	4.4114*E* − 01	**1.7940*E*** + **01**	−4.0649*E* + 00	**4.5717*E*** + **00**
F14 *p* value	**1.3970*E* − 09**	**1.1918*E* − 18**	**5.8521*E* − 05**	1.0000*E* + 00	8.7069*E* − 01	1.0000*E* + 00
*t*-value	**8.4209*E*** + **00**	**1.9727*E*** + **01**	**4.4485*E*** + **00**	−7.6068*E* + 00	−1.1523*E* + 00	−6.1445*E* + 00
F15 *p* value	**4.4169*E* − 02**	0.0000*E* + 00	1.0351*E* − 01	**1.4225*E* − 28**	**4.0579*E* − 02**	1.6279*E* − 01
*t*-value	**1.7636*E*** + **00**	6.5535*E* + 04	1.2907*E* + 00	**4.4596*E*** + **01**	**1.8069*E*** + **00**	1.0000*E* + 00
F16 *p* value	**2.2146*E* − 35**	**1.8681*E* − 02**	**1.6670*E* − 26**	**9.4398*E* − 06**	**4.4541*E* − 03**	**2.0580*E* − 11**
*t*-value	**7.8793*E*** + **01**	**2.4917*E*** + **00**	**3.8667*E*** + **01**	**5.3557*E*** + **00**	**3.0840*E*** + **00**	**−1.0521*E*** + **01**
F17 *p* value	**1.6862*E* − 14**	**2.8856*E* − 14**	**2.9742*E* − 11**	**2.4646*E* − 17**	**1.4025*E* − 15**	**2.7998*E* − 05**
*t*-value	**1.4084*E*** + **01**	**1.3789*E*** + **01**	**1.0355*E*** + **01**	**1.8085*E*** + **01**	**1.5515*E*** + **01**	**4.9645*E*** + **00**
F18 *p* value	**8.1734*E* − 40**	**6.2243*E* − 13**	**1.5126*E* − 13**	**2.4389*E* − 26**	**7.4395*E* − 14**	**2.6112*E* − 12**
*t*-value	**1.1216*E*** + **02**	**1.2186*E*** + **01**	**1.2907*E*** + **01**	**3.8153*E*** + **01**	**1.3279*E*** + **01**	**1.1485*E*** + **01**
F19 *p* value	**7.8659*E* − 16**	**6.3716*E* − 16**	**2.5304*E* − 29**	**7.3198*E* − 09**	**9.1664*E* − 03**	**5.7997*E* − 11**
*t*-value	**1.5863*E*** + **01**	**1.5992*E*** + **01**	**4.8529*E*** + **01**	**8.0358*E*** + **00**	**2.7924*E*** + **00**	**−1.0057*E*** + **01**
F20 *p* value	2.0538*E* − 01	1.0945*E* − 01	3.5879*E* − 01	**1.5016*E* − 02**	**4.2555*E* − 02**	5.8238*E* − 01
*t*-value	1.2955*E* + 00	1.6514*E* + 00	9.3247*E* − 01	**2.5855*E*** + **00**	**2.1214*E*** + **00**	5.5614*E* − 01
F21 *p* value	**8.3632*E* − 19**	**9.8736*E* − 13**	**1.4395*E* − 02**	**2.9524*E* − 12**	**2.6133*E* − 10**	**2.2364*E* − 05**
*t*-value	**2.0503*E*** + **01**	**1.1958*E*** + **01**	**−2.6035*E*** + **00**	**1.1426*E*** + **01**	**9.4036*E*** + **00**	**−5.0453*E*** + **00**
F22 *p* value	**1.0184*E* − 22**	**4.1524*E* − 08**	**1.6168*E* − 20**	**2.1637*E* − 14**	**2.7111*E* − 07**	2.3769*E* − 01
*t*-value	**2.8405*E*** + **01**	**7.3599*E*** + **00**	**2.3678*E*** + **01**	**1.3947*E*** + **01**	**6.6517*E*** + **00**	1.2057*E* + 00
F23 *p* value	**7.7098*E* − 25**	**1.6951*E* − 15**	**2.7714*E* − 22**	**1.9645*E* − 07**	**1.3576*E* − 10**	**1.3455*E* − 06**
*t*-value	**3.3782*E*** + **01**	**1.5402*E*** + **01**	**2.7407*E*** + **01**	**6.7718*E*** + **00**	**9.6849*E*** + **00**	**6.0616*E*** + **00**
F24 *p* value	**2.3504*E* − 11**	**1.6781*E* − 04**	**1.8959*E* − 05**	**1.0796*E* − 19**	**1.3665*E* − 09**	6.1715*E* − 02
*t*-value	**1.0461*E*** + **01**	**4.3178*E*** + **00**	**5.1047*E*** + **00**	**2.2099*E*** + **01**	**8.7120*E*** + **00**	−1.9435*E* + 00
F25 *p* value	**3.0199*E* − 11**	**3.3384*E* − 11**	**1.4110*E* − 09**	5.0912*E* − 06	**2.0152*E* − 08**	**1.3272*E* − 02**
*t*-value	**6.6456*E*** + **00**	**6.6308*E*** + **00**	**6.0542*E*** + **00**	−4.5610*E* + 00	**5.6107*E*** + **00**	**2.4764*E*** + **00**
F26 *p* value	**3.0199*E* − 11**	**3.0199*E* − 11**	**3.0199*E* − 11**	**3.0199*E* − 11**	**3.0199*E* − 11**	**3.0199*E* − 11**
*t*-value	**6.6456*E*** + **00**	**6.6456*E*** + **00**	**6.6456*E*** + **00**	**6.6456*E*** + **00**	**6.6456*E*** + **00**	**6.6456*E*** + **00**
F27 *p* value	**3.0199*E* − 11**	**3.0199*E* − 11**	**3.0199*E* − 11**	**3.0199*E* − 11**	**3.0199*E* − 11**	**8.4848*E* − 09**
*t*-value	**6.6456*E*** + **00**	**6.6456*E*** + **00**	**6.6456*E*** + **00**	**6.6456*E*** + **00**	**6.6456*E*** + **00**	**5.7585*E*** + **00**
F28 *p* value	**3.0199*E* − 11**	**1.3289*E* − 10**	**3.3384*E* − 11**	**3.0199*E* − 11**	**3.0199*E* − 11**	1.4532*E* − 01
*t*-value	**6.6456*E*** + **00**	**6.4238*E*** + + **00**	**6.6308*E*** + **00**	**6.6456*E*** + **00**	**6.6456*E*** + **00**	−1.4563*E* + 00
F29 *p* value	**3.0199*E* − 11**	**3.0199*E* − 11**	**3.0199*E* − 11**	**3.0199*E* − 11**	**3.0199*E* − 11**	**5.0922*E* − 08**
*t*-value	**6.6456*E*** + **00**	**6.6456*E*** + **00**	**6.6456*E*** + **00**	**6.6456*E*** + **00**	**6.6456*E*** + **00**	**5.4481*E*** + **00**
F30 *p* value	4.6159*E* − 10	1.6285*E* − 02	**8.1975*E* − 07**	**8.4848*E* − 09**	**6.3560*E* − 05**	**7.2208*E* − 06**
*t*-value	−6.2316*E* + 00	−2.4025*E* + 00	**4.9306*E*** + **00**	**5.7585*E*** + **00**	**3.9992*E*** + **00**	**4.4871*E*** + **00**
**B/N/W**	**19/10/1**	**17/12/1**	**21/9/0**	**23/6/1**	**25/5/0**	**17/13/0**

The article "An Evolutionary Frog Leaping Algorithm for Global Optimization Problems and Applications" was published in 2021. Journal: Comput Intell Neurosci.

**Table 6:** *T*−test for comparison results with EFLA and other algorithms.

Func	SFLA	SSA	CMAES	SCA	AAA	GWO
F1 *p* value	1.1970*E* − 01	**4.7988*E* − 25**	**2.5751*E* − 29**	1.3152*E* − 01	**2.9482*E* − 04**	0.0000*E* + 00
*t*-value	1.2012*E* + 00	**3.3521*E*** + **01**	**4.7340*E*** + **01**	1.1414*E* + 00	**3.8566*E*** + **00**	6.5535*E* + 04
F2 *p* value	1.5116*E* − 01	**2.6757*E* − 22**	**7.1377*E* − 30**	1.6279*E* − 01	**1.8179*E* − 03**	1.0000*E* + 00
*t*-value	1.0501*E* + 00	**2.6769*E*** + **01**	**4.9508*E*** + **01**	1.0000*E* + 00	**3.1642*E*** + **00**	6.5535*E* + 04
F3 *p* value	**4.4555*E* − 13**	**5.2131*E* − 03**	**2.0376*E* − 27**	1.4702*E* − 01	**1.5207*E* − 08**	9.8639*E* − 02
*t*-value	**1.2008*E*** + **01**	**2.7391*E*** + **00**	**4.0626*E*** + **01**	1.0686*E* + 00	**7.4795*E*** + **00**	1.3196*E* + 00
F4 *p* value	1.0803*E* − 01	**3.7450*E* − 14**	**2.0769*E* − 18**	**4.5253*E* − 02**	**3.7838*E* − 16**	1.0000*E* + 00
*t*-value	1.2646*E* + 00	**1.3276*E*** + **01**	**1.9325*E*** + **01**	**1.7511*E*** + **00**	**1.5887*E*** + **01**	−7.7421*E* + 00
F5 *p* value	**1.2480*E* − 15**	**2.6583*E* − 22**	**7.7173*E* − 22**	1.6279*E* − 01	1.6279*E* − 01	**1.5887*E* − 02**
*t*-value	**1.5173*E*** + **01**	**2.6776*E*** + **01**	**2.5771*E*** + **01**	1.0000*E* + 00	1.0000*E* + 00	**2.2562*E*** + **00**
F6 *p* value	**3.1631*E* − 03**	**7.9655*E* − 12**	**1.3084*E* − 59**	**7.1294*E* − 04**	**8.6649*E* − 14**	**4.3506*E* − 06**
*t*-value	**2.9436*E*** + **00**	**1.0638*E*** + **01**	**5.2787*E*** + **02**	**3.5254*E*** + **00**	**1.2836*E*** + **01**	**5.3851*E*** + **00**
F7 *p* value	**3.3383*E* − 08**	**1.6255*E* − 06**	**1.4964*E* − 02**	**−**	**−**	1.6279*E* − 01
*t*-value	**7.1786*E*** + **00**	**5.7407*E*** + **00**	**2.2833*E*** + **00**	**−**	**−**	1.0000*E* + 00
F8 *p* value	**4.9354*E* − 05**	**1.0092*E* − 03**	1.0000*E* + 00	**1.3414*E* − 25**	9.9993*E* − 01	**7.5857*E* − 26**
*t*-value	**4.5102*E*** + **00**	**3.3927*E*** + **00**	−8.6414*E* + 01	**3.5064*E*** + **01**	−4.3746*E* + 00	**3.5776*E*** + **01**
F9 *p* value	9.7187*E* − 01	**1.7840*E* − 06**	9.5712*E* − 01	**9.1216*E* − 13**	9.8253*E* − 01	9.6146*E* − 01
*t*-value	−1.9886*E* + 00	**5.7071*E*** + **00**	−1.7788*E* + 00	**1.1658*E*** + **01**	−2.2127*E* + 00	−1.8331*E* + 00
F10 *p* value	**7.1766*E* − 13**	**2.0033*E* − 20**	**2.3274*E* − 08**	**—**	**—**	−
*t*-value	**1.1774*E*** + **01**	**2.2911*E*** + **01**	**7.3162*E*** + **00**	**—**	**—**	−
F11 *p* value	**2.2041*E* − 12**	1.6271*E* − 01	**7.4411*E* − 28**	**7.4421*E* − 03**	**2.6435*E* − 05**	**4.7099*E* − 02**
*t*-value	**1.1235*E*** + **01**	1.0003*E* + 00	**4.2086*E*** + **01**	**2.5893*E*** + **00**	**4.7356*E*** + **00**	**1.7303*E*** + **00**
F12 *p* value	**3.1827*E* − 02**	**4.3936*E* − 12**	**7.8558*E* − 04**	9.9882*E* − 01	7.4249*E* − 01	9.9882*E* − 01
*t*-value	**1.9284*E*** + **00**	**1.0912*E*** + **01**	**3.4885*E*** + **00**	−3.3312*E* + 00	−6.5912*E* − 01	−3.3312*E* + 00
F13 *p* value	**7.7454*E* − 19**	**1.0832*E* − 18**	**1.9836*E* − 16**	1.0000*E* + 00	**2.9930*E* − 16**	9.9998*E* − 01
*t*-value	**2.0043*E*** + **01**	**1.9796*E*** + **01**	**1.6283*E*** + **01**	−1.6155*E* + 01	**1.6030*E*** + **01**	−4.7848*E* + 00
F14 *p* value	3.4856*E* − 01	1.0000*E* + 00	1.0000*E* + 00	**5.6018*E* − 05**	1.0000*E* + 00	**1.2412*E* − 36**
*t*-value	3.9309*E* − 01	−7.6068*E* + 00	−7.6068*E* + 00	**4.4644*E*** + **00**	−7.6068*E* + 00	**8.4996*E*** + **01**
F15 *p* value	1.5976*E* − 01	**1.1120*E* − 16**	**1.1595*E* − 08**	1.6279*E* − 01	**3.5115*E* − 04**	1.0000*E* + 00
*t*-value	1.0128*E* + 00	**1.6646*E*** + **01**	**7.5843*E*** + **00**	1.0000*E* + 00	**3.7916*E*** + **00**	6.5535*E* + 04
F16 p value	**1.6843*E* − 15**	3.9318*E* − 01	**6.3185*E* − 11**	**4.6127*E* − 27**	**2.0380*E* − 02**	**1.0156*E* − 08**
*t*-value	**1.5406*E*** + **01**	8.6677*E* − 01	**−1.0019*E*** + **01**	**4.0450*E*** + **01**	**−2.4538*E*** + **00**	**7.9065*E*** + **00**
F17 *p* value	**3.3232*E* − 25**	**1.9599*E* − 11**	2.2203*E* − 09	**9.5786*E* − 17**	**2.9649*E* − 08**	**1.1868*E* − 12**
*t*-value	**3.4801*E*** + **01**	**1.0543*E*** + **01**	−8.5140*E* + 00	**1.7185*E*** + **01**	**7.4894*E*** + **00**	**1.1867*E*** + **01**
F18 *p* value	**3.2445*E* − 28**	**2.0759*E* − 11**	4.1154*E* − 06	**6.9813*E* − 26**	**6.8464*E* − 20**	**2.4283*E* − 11**
*t*-value	**4.4391*E*** + **01**	**1.0517*E*** + **01**	−5.6554*E* + 00	**3.6768*E*** + **01**	**2.2469*E*** + **01**	**1.0446*E*** + **01**
F19 *p* value	**8.7173*E* − 24**	**6.9426*E* − 32**	6.1959*E* − 02	**1.4268*E* − 15**	3.5211*E* − 06	**9.0159*E* − 11**
*t*-value	**3.1002*E*** + **01**	**5.9593*E*** + **01**	1.9416*E* + 00	**1.5504*E*** + **01**	−5.7118*E* + 00	**9.8630*E*** + **00**
F20 *p* value	**1.2367*E* − 02**	4.6527*E* − 01	**4.6523*E* − 02**	3.1829*E* − 01	5.1373*E* − 01	2.3344*E* − 01
*t*-value	**2.6677*E*** + **00**	−7.3997*E* − 01	**2.0795*E*** + **00**	1.0154*E* + 00	6.6115*E* − 01	1.2169*E* + 00
F21 *p* value	**4.7609*E* − 15**	**2.8266*E* − 07**	**7.4429*E* − 17**	**2.0334*E* − 21**	**2.2252*E* − 03**	**1.1693*E* − 07**
*t*-value	**1.4798*E*** + **01**	**6.6362*E*** + **00**	**1.7350*E*** + **01**	**2.5517*E*** + **01**	**3.3552*E*** + **00**	**6.9665*E*** + **00**
F22 *p* value	**4.5203*E* − 24**	1.7111*E* − 04	6.8284*E* − 10	**4.7594*E* − 21**	5.1359*E* − 01	**3.0037*E* − 11**
*t*-value	**3.1732*E*** + **01**	−4.3107*E* + 00	−8.9989*E* + 00	**2.4747*E*** + **01**	6.6138*E* − 01	**1.0350*E*** + **01**
F23 *p* value	**1.5634*E* − 06**	**3.1673*E* − 07**	**7.1356*E* − 11**	**2.3312*E* − 25**	**2.8253*E* − 04**	**1.6599*E* − 19**
*t*-value	**6.0068*E*** + **00**	**6.5939*E*** + **00**	**9.9656*E*** + **00**	**3.5238*E*** + **01**	**4.1277*E*** + **00**	**2.1755*E*** + **01**
F24 *p* value	**6.3207*E* − 07**	**1.4501*E* − 04**	**2.2210*E* − 06**	**1.3569*E* − 15**	**3.9789*E* − 07**	**4.9996*E* − 04**
*t*-value	**6.3385*E*** + **00**	**4.3708*E*** + **00**	**5.8790*E*** + **00**	**1.5534*E*** + **01**	**6.5093*E*** + **00**	**3.9177*E*** + **00**
F25 *p* value	**6.9125*E* − 04**	**1.8500*E* − 08**	**8.1527*E* − 11**	**3.0199*E* − 11**	1.5292*E* − 05	**6.9125*E* − 04**
*t*-value	**3.3930*E*** + **00**	**5.6255*E*** + **00**	**6.4978*E*** + **00**	**6.6456*E*** + **00**	−4.3244*E* + 00	**3.3930*E*** + **00**
F26 *p* value	**3.0199*E* − 11**	**3.0199*E* − 11**	**3.6459*E* − 08**	**3.0199*E* − 11**	**3.0199*E* − 11**	**3.0199*E* − 11**
*t*-value	**6.6456*E*** + **00**	**6.6456*E*** + **00**	**5.5072*E*** + **00**	**6.6456*E*** + **00**	**6.6456*E*** + **00**	**6.6456*E*** + **00**
F27 *p* value	**3.0199*E* − 11**	**3.0199*E* − 11**	**4.3531*E* − 05**	**3.0199*E* − 11**	**6.7362*E* − 06**	**3.0199*E* − 11**
*t*-value	**6.6456*E*** + **00**	**6.6456*E*** + **00**	**4.0879*E*** + **00**	**6.6456*E*** + **00**	**4.5019*E*** + **00**	**6.6456*E*** + **00**
F28 *p* value	**3.0199*E* − 11**	**3.0199*E* − 11**	**3.4742*E* − 10**	**3.0199*E* − 11**	**3.0199*E* − 11**	**3.0199*E* − 11**
*t*-value	**6.6456*E*** + **00**	**6.6456*E*** + **00**	**6.2760*E*** + **00**	**6.6456*E*** + **00**	**6.6456*E*** + **00**	**6.6456*E*** + **00**
F29 *p* value	**3.0199*E* − 11**	**3.0199*E* − 11**	**6.1210*E* − 10**	**3.0199*E* − 11**	**3.0199*E* − 11**	**3.0199*E* − 11**
*t*-value	**6.6456*E*** + **00**	**6.6456*E*** + **00**	**6.1873*E*** + **00**	**6.6456*E*** + **00**	**6.6456*E*** + **00**	**6.6456*E*** + **00**
F30 *p* value	**1.4067*E* − 04**	**6.0658*E* − 11**	**1.2541*E* − 07**	5.2014*E* − 01	**2.5974*E* − 05**	**8.8411*E* − 07**
*t*-value	**3.8070*E*** + **00**	**6.5421*E*** + **00**	**5.2854*E*** + **00**	−6.4312*E* − 01	**4.2062*E*** + **00**	**−4.9158*E*** + **00**
**B/N/W**	**24/6/0**	**25/4/1**	**24/3/3**	**22/8/0**	**20/82**	**19/11/0**

The article "An Evolutionary Frog Leaping Algorithm for Global Optimization Problems and Applications" was published in 2021. Journal: Comput Intell Neurosci.

**Table 7:** Wilcoxon signed-rank test for comparison results of EFLA and other algorithms.

Func	LAPO	TSQPSO	WQPSO	GbABC	NNA	SaDE	SFLA	SSA	CMAES	SCA	AAA	GWO
F1	+	+	+	+	+	+	+	+	+	+	+	+
F2	+	+	+	+	+	+	+	+	+	+	+	−
F3	+	+	+	+	+	+	+	+	+	+	+	+
F4	−	−	−	+	−	+	+	+	+	+	+	−
F5	=	+	+	=	+	=	+	+	+	+	+	+
F6	+	−	−	+	+	+	+	+	+	+	+	+
F7	+	+	+	=	+	+	+	+	+	=	=	+
F8	+	+	+	−	+	+	+	+	−	+	−	+
F9	+	−	−	−	−	−	−	+	−	+	−	−
F10	=	=	=	=	+	+	+	+	+	=	=	=
F11	+	+	+	+	+	+	+	+	+	+	+	+
F12	−	+	+	+	+	−	+	+	+	−	−	−
F13	−	−	+	+	−	+	+	+	+	−	+	−
F14	+	+	+	−	−	−	+	−	−	+	−	+
F15	+	+	+	+	+	+	+	+	+	+	+	−
F16	+	+	+	+	+	−	+	+	−	+	−	+
F17	+	+	+	+	+	+	+	+	−	+	+	+
F18	+	+	+	+	+	+	+	+	−	+	+	+
F19	+	+	+	+	+	−	+	+	+	+	−	+
F20	+	+	+	+	+	+	+	−	+	+	+	+
F21	+	+	−	+	+	−	+	+	+	+	+	+
F22	+	+	+	+	+	+	+	−	−	+	+	+
F23	+	+	+	+	+	+	+	+	+	+	+	+
F24	+	+	+	+	+	−	+	+	+	+	+	+
F25	+	+	+	−	+	+	+	+	+	+	−	+
F26	+	+	+	+	+	+	+	+	+	+	+	+
F27	+	+	+	+	+	−	+	+	+	+	+	+
F28	+	+	+	+	+	+	+	+	+	+	+	+
F29	+	+	+	+	+	+	+	+	+	+	+	+
F30	−	−	+	+	+	+	+	+	+	−	+	−
Total												
w/e/l	**24/2/4**	**24/1/5**	**25/1/4**	**23/3/4**	**26/0/4**	**21/1/8**	**29/0/1**	**27/0/3**	**23/0/7**	**25/2/3**	**21/2/7**	**22/1/7**
*p* value	**1.07*e* − 004**	**1.53*e* − 003**	**7.14*e* − 004**	**1.28*e* − 003**	**2.83*e* − 004**	**2.00*e* − 002**	**5.73*e* − 006**	**6.31*e* − 005**	**2.95*e* − 003**	**8.97*e* − 005**	**1.39*e* − 002**	**1.32*e* − 003**
*z*−value	**−3.8737**	**−3.1678**	**−3.3840**	**−3.2195**	**−3.6303**	**−2.3245**	**−4.5358**	**−4.0006**	**−2.9721**	**−3.9167**	**−2.4593**	**−3.2110**

**Table 8:** Friedman test for EFLA and other algorithms.

Order	Algorithm	Averages ranks
**1**	**EFLA**	**3.12**
2	SaDE	5.12
3	AAA	5.50
4	TSQPSO	6.35
5	WQPSO	6.48
6	GWO	6.82
7	CMAES	7.00
8	SSA	7.77
9	NNA	7.93
10	GbABC	7.98
11	LAPO	8.30
12	SFLA	9.27
13	SCA	9.37

**Table 9:** Statistical value of the Friedman test for EFLA and other algorithms.

Method	Statistical value	*P* value
Friedman test	72.8290	9.43E−11

**Table 10:** Comparison results for 13 algorithms (*D* = 100).

Algorithms	F1	R	F3	R	F20	R	F23	R	F28	R	F29	R
AAA mean	1.1125E−79	**6**	4.4886*E* + 03	**10**	**2.1242*E*** + **01**	**1**	**1.4474*E*** + **04**	**1**	7.1266*E* + 04	**10**	2.5430*E* + 06	**6**
Std.	2.5740E−79		1.4235*E* + 03		**6.0063*E* − 02**		**1.2360*E* + 03**		1.7915*E* + 04		9.6863*E* + 05	
**EFLA** mean	**6.6252*E* − 286**		**6.0290*E* − 07**		2.1253*E* + 01		1.4736*E* + 04		**8.4302*E*** + **02**		**1.5399*E*** + **05**	
Std.	**0.0000*E*** + **00**		**1.4203*E* − 06**		3.4012E−02		2.4380*E* + 03		**1.4322*E*** + **02**		**7.2197*E*** + **04**	
GWO mean	**0.0000*E*** + **00**	**1**	5.8937E−03	**4**	2.1277*E* + 01	**4**	2.9645*E* + 04	**10**	1.0410*E* + 04	**7**	1.1259*E* + 07	**10**
Std.	**0.0000*E*** + **00**		2.0000E−02		4.8661E−02		3.7559*E* + 03		6.0506*E* + 03		4.2230*E* + 06	
**EFLA** mean	6.6252E−286		**6.0290*E* − 07**		**2.1253*E*** + **01**		**1.4736*E*** + **04**		**8.4302*E*** + **02**		**1.5399*E*** + **05**	
Std.	0.0000*E* + 00		**1.4203*E* − 06**		**3.4012*E* − 02**		**2.4380*E*** + **03**		**1.4322*E*** + **02**		**7.2197*E*** + **04**	
CMAES mean	1.3759E−28	**8**	**8.7795*E* − 27**	**2**	2.1278*E* + 01	**5**	1.6447*E* + 04	**6**	8.7535*E* + 02	**2**	**3.6520*E*** + **03**	**1**
Std.	6.7881E−30		**6.1501*E* − 28**		5.3762E−02		1.3676*E* + 03		1.6156*E* + 02		**5.4436*E*** + **02**	
**EFLA** mean	**6.6252*E* − 286**		6.0290E−07		**2.1253*E*** + **01**		**1.4736*E*** + **04**		**8.4302*E*** + **02**		1.5399*E* + 05	
Std.	**0.0000*E*** + **00**		1.4203E−06		**3.4012*E* − 02**		**2.4380*E*** + **03**		**1.4322*E*** + **02**		7.2197*E* + 04	
LAPO mean	**0.0000*E*** + **00**	**1**	**2.8293*E* − 32**	**1**	2.1293*E* + 01	**8**	3.0373*E* + 04	**11**	7.6865*E* + 05	**13**	3.7556*E* + 08	**13**
Std.	**0.0000*E*** + **00**		**1.5481*E* − 31**		2.7631E−02		6.1967*E* + 02		1.5186*E* + 05		7.3274*E* + 07	
**EFLA** mean	6.6252E−286		6.0290E−07		**2.1253*E*** + **01**		**1.4736*E*** + **04**		**8.4302*E*** + **02**		**1.5399*E*** + **05**	
Std.	0.0000*E* + 00		1.4203E−06		**3.4012*E* − 02**		**2.4380*E*** + **03**		**1.4322*E*** + **02**		**7.2197*E*** + **04**	
SFLA mean	1.4904E−13	**11**	3.0880*E* + 02	**9**	2.1303*E* + 01	**10**	1.6551*E* + 04	**7**	1.0833*E* + 04	**8**	3.2197*E* + 06	**7**
Std.	8.0803E−13		5.9743*E* + 01		2.2014E−02		2.0443*E* + 03		1.4502*E* + 03		5.3386*E* + 05	
**EFLA** mean	**6.6252*E* − 286**		**6.0290*E* − 07**		**2.1253*E*** + **01**		**1.4736*E*** + **04**		**8.4302*E*** + **02**		**1.5399*E*** + **05**	
Std.	**0.0000*E*** + **00**		**1.4203*E* − 06**		**3.4012*E* − 02**		**2.4380*E*** + **03**		**1.4322*E*** + **02**		**7.2197*E*** + **04**	
NNA mean	5.1299E−17	**9**	3.6852*E* + 00	**5**	2.1283*E* + 01	**6**	1.9107*E* + 04	**8**	1.2615*E* + 04	**9**	7.7348*E* + 06	
Std.	1.2987E−16		1.4683*E* + 01		3.6170E−02		1.5868*E* + 03		6.1335*E* + 03		2.5688*E* + 06	
**EFLA** mean	**6.6252*E* − 286**		**6.0290*E* − 07**		**2.1253*E*** + **01**		**1.4736*E*** + **04**		**8.4302*E*** + **02**		**1.5399*E*** + **05**	**11**
Std.	**0.0000*E*** + **00**		**1.4203*E* − 06**		**3.4012*E* − 02**		**2.4380*E*** + **03**		**1.4322*E* + 02**		**7.2197*E*** + **04**	
GbABC mean	1.5196E−15	**10**	4.5842*E* + 04	**12**	2.1308*E* + 01	**13**	1.6237*E* + 04	**5**	1.2516*E* + 05	**11**	1.1578*E* + 07	
Std.	1.2251E−16		7.5077*E* + 03		2.4901E−02		9.0027*E* + 02		2.8233*E* + 04		3.5576*E* + 06	
**EFLA** mean	**6.6252*E* − 286**		**6.0290*E* − 07**		**2.1253*E*** + **01**		**1.4736*E*** + **04**		**8.4302*E*** + **02**		**1.5399*E*** + **05**	
Std.	**0.0000*E*** + **00**		**1.4203*E* − 06**		**3.4012*E* − 02**		**2.4380*E*** + **03**		**1.4322*E*** + **02**		**7.2197*E*** + **04**	
SSA mean	2.1980E−51	**7**	2.3486*E* + 02	**8**	**2.1252*E*** + **01**	**2**	**1.4561*E*** + **04**	**2**	1.7156*E* + 03	**5**	9.2387*E* + 05	**4**
Std.	2.7362E−52		7.1058*E* + 01		**4.5617*E* − 02**		**1.5796*E*** + **03**		3.5664*E* + 02		4.4898*E* + 05	
**EFLA** mean	**6.6252*E* − 286**		**6.0290*E* − 07**		2.1253*E* + 01		1.4736*E* + 04		**8.4302*E*** + **02**		**1.5399*E*** + **05**	
Std.	**0.0000*E*** + **00**		**1.4203*E* − 06**		3.4012E−02		2.4380*E* + 03		**1.4322*E*** + **02**		**7.2197*E*** + **04**	
SCA mean	1.6964*E* + 01	**12**	7.6202*E* + 04	**13**	2.1304*E* + 01	**11**	3.0799*E* + 04	**13**	1.3059*E* + 05	**12**	7.6041*E* + 07	**12**
Std.	9.2820*E* + 01		2.1699*E* + 04		2.6376E−02		4.6271*E* + 02		3.4908*E* + 04		2.1585*E* + 07	
**EFLA** mean	**6.6252*E* − 286**		**6.0290*E* − 07**		**2.1253*E*** + **01**		**1.4736*E*** + **04**		**8.4302*E*** + **02**		**1.5399*E*** + **05**	
Std.	**0.0000*E*** + **00**		**1.4203*E* − 06**		**3.4012*E* − 02**		**2.4380*E*** + **03**		**1.4322*E*** + **02**		**7.2197*E*** + **04**	
TSQPSO mean	2.0134E−244	**3**	2.3121*E* + 02	**7**	2.1287*E* + 01	**7**	2.8306*E* + 04	**9**	1.1922*E* + 03	**3**	3.2510*E* + 06	**8**
Std.	0.0000*E* + 00		9.2601*E* + 01		4.0094E−02		1.4779*E* + 03		3.7968*E* + 02		1.1347*E* + 06	
**EFLA** mean	**6.6252*E* − 286**		**6.0290*E* − 07**		**2.1253*E*** + **01**		**1.4736*E*** + **04**		**8.4302*E*** + **02**		**1.5399*E*** + **05**	
Std.	**0.0000*E*** + **00**		**1.4203*E* − 06**		**3.4012*E* − 02**		**2.4380*E*** + **03**		**1.4322*E*** + **02**		**7.2197*E*** + **04**	
WQPSO mean	3.1583E−88	**5**	1.1209*E* + 04	**11**	2.1296*E* + 01	**9**	3.0533*E* + 04	**12**	1.3082*E* + 03	**4**	3.6247*E* + 06	**9**
Std.	8.1474E−88		3.9403*E* + 03		3.6636E−02		4.3334*E* + 02		3.1719*E* + 02		1.4590*E* + 06	
**EFLA** mean	**6.6252*E* − 286**		**6.0290*E* − 07**		**2.1253*E*** + **01**		**1.4736*E*** + **04**		**8.4302*E*** + **02**		**1.5399*E*** + **05**	
Std.	**0.0000*E*** + **00**		**1.4203*E* − 06**		**3.4012*E* − 02**		**2.4380*E*** + **03**		**1.4322*E*** + **02**		**7.2197*E*** + **04**	
SaDE mean	6.7961E−94	**4**	4.7911*E* + 00	**6**	2.1305*E* + 01	**12**	1.4912*E* + 04	**4**	6.7720*E* + 03	**6**	2.9824*E* + 05	**3**
Std.	3.1491E−93		2.0130*E* + 00		2.8644E−02		2.0069*E* + 03		2.9429*E* + 03		1.0970*E* + 05	
**EFLA** mean	**6.6252*E* − 286**	**2**	**6.0290*E* − 07**	**3**	**2.1253*E*** + **01**	**3**	**1.4736*E*** + **04**	**3**	**8.4302*E*** + **02**	**1**	**1.5399*E*** + **05**	**2**
Std.	**0.0000*E*** + **00**		**1.4203*E* − 06**		**3.4012*E* − 02**		**2.4380*E*** + **03**		**1.4322*E*** + **02**		**7.2197*E*** + **04**	

The article "An Evolutionary Frog Leaping Algorithm for Global Optimization Problems and Applications" was published in 2021. Journal: Comput Intell Neurosci.

**Table 11:** Friedman test for EFLA and other algorithms.

Order	Algorithm	Averages ranks
**1**	**EFLA**	**2.50**
2	CMAES	4.17
3	SSA	4.83
4	AAA	5.67
5	SaDE	6.00
6	GWO	6.08
7	TSQPSO	6.17
8	NNA	7.83
9	LAPO	7.92
10	WQPSO	8.33
11	SFLA	8.67
12	GbABC	10.50
13	SCA	12.33

**Table 12:** Statistical value of the Friedman test for EFLA and other algorithms.

Method	Statistical value	*p* value
Friedman test	33.273	0.001

**Table 13:** Comparison results of EFLA with different parameters.

Func	EFLA01	R	EFLA02	R	EFLA03	R	EFLA04	R	EFLA05	R	EFLA06	R
	(*m* = 2, *n* = 10)		(*m* = 4, *n* = 5)		(*m* = 5, *n* = 4)		(*m* = 10, *n* = 2)		(*m* = 6, *n* = 5)		(*m* = 5, *n* = 8	
F1 mean	**0.0000 *E*** + **00**	**1**	**0.0000 *E*** + **00**	**1**	**0.0000 *E*** + **00**	**1**	**0.0000 *E*** + **00**	**1**	**1.9097*E* − 232**	**2**	6.2681*E* − 183	**3**
Std.	**0.0000 *E*** + **00**		**0.0000 *E*** + **00**		**0.0000 *E*** + **00**		**0.0000 *E*** + **00**		**0.0000 *E*** + **00**		0.0000 *E* + 00	
F2 mean	**0.0000 *E*** + **00**	**1**	**0.0000 *E*** + **00**	**1**	**0.0000 *E*** + **00**	**1**	**0.0000 *E*** + **00**	**1**	**3.3520*E* − 233**	**2**	9.5917*E* − 185	**3**
Std.	**0.0000 *E*** + **00**		**0.0000 *E*** + **00**		**0.0000 *E*** + **00**		**0.0000 *E*** + **00**		**0.0000 *E*** + **00**		0.0000 *E* + 00	
F3 mean	**1.7978*E* − 40**	**1**	8.0141*E* − 37	**2**	1.1384*E* − 36	**3**	1.4129*E* − 30	**6**	3.3911*E* − 34	**4**	8.8138*E* − 31	**5**
Std.	**5.7417*E* − 40**		4.0605*E* − 36		4.5785*E* − 36		6.5852*E* − 30		1.5866*E* − 33		4.5372*E* − 30	
F4 mean	1.7724*E* − 03	**5**	1.6305*E* − 03	**3**	1.3683*E* − 03	**2**	**1.2968*E* − 03**	**1**	1.7149*E* − 03	**4**	2.0379*E* − 03	**7**
Std.	7.0959*E* − 04		8.2673*E* − 04		6.7566*E* − 04		**6.9047*E* − 04**		1.0814*E* − 03		5.9870*E* − 04	
F5 mean	**0.0000 *E*** + **00**	**1**	**0.0000 *E*** + **00**	**1**	**0.0000 *E*** + **00**	**1**	**0.0000 *E*** + **00**	**1**	**0.0000 *E*** + **00**	**1**	4.3163*E* − 01	**3**
Std.	**0.0000 *E*** + **00**		**0.0000 *E*** + **00**		**0.0000 *E*** + **00**		**0.0000 *E*** + **00**		**0.0000 *E*** + **00**		2.3641 *E* + 00	
F6 mean	8.7634*E* − 15	**9**	7.3423*E* − 15	**5**	6.8686*E* − 15	**2**	**5.4475*E* − 15**	**1**	7.2239*E* − 15	**4**	7.5791*E* − 15	**6**
Std.	3.0566*E* − 15		1.2973*E* − 15		9.0135*E* − 16		**1.8027*E* − 15**		1.4703*E* − 15		1.8027*E* − 15	
F7 mean	**0.0000 *E*** + **00**	**1**	**0.0000 *E*** + **00**	**1**	**0.0000 *E*** + **00**	**1**	**0.0000 *E*** + **00**	**1**	**0.0000 *E*** + **00**	**1**	**0.0000 *E*** + **00**	**1**
Std.	**0.0000 *E*** + **00**		**0.0000 *E*** + **00**		**0.0000 *E*** + **00**		**0.0000 *E*** + **00**		**0.0000 *E*** + **00**		**0.0000 *E*** + **00**	
F8 mean	2.0006 *E* + 01	**9**	2.1241 *E* + 01	**10**	2.1404 *E* + 01	**11**	2.1583 *E* + 01	**12**	1.9977 *E* + 01	**8**	1.5395 *E* + 01	**3**
Std.	8.9636*E* − 01		7.0601*E* − 01		3.0286*E* − 01		5.8636*E* − 01		7.8322*E* − 01		1.3703 *E* + 00	
F9 mean	7.6067*E* − 02	**10**	1.1415*E* − 01	**11**	3.1100*E* − 02	**4**	7.6015*E* − 02	**8**	4.4920*E* − 02	**6**	1.4528*E* − 01	**12**
Std.	2.7508*E* − 01		2.6342*E* − 01		5.5459*E* − 02		1.5139*E* − 01		1.1119*E* − 01		3.0329*E* − 01	
F10 mean	7.4015*E* − 18	**2**	**0.0000 *E*** + **00**	**1**	**0.0000 *E*** + **00**	**1**	**0.0000 *E*** + **00**	**1**	**0.0000 *E*** + **00**	**1**	**0.0000 *E*** + **00**	**1**
Std.	4.0540*E* − 17		**0.0000 *E*** + **00**		**0.0000 *E*** + **00**		**0.0000 *E*** + **00**		**0.0000 *E*** + **00**		**0.0000 *E*** + **00**	
F11 mean	**4.3004*E* − 107**	**1**	5.4823*E* − 107	**2**	2.3415*E* − 106	**3**	6.4680*E* − 99	**4**	4.0066*E* − 75	**5**	5.3763*E* − 61	**6**
Std.	**1.4184*E* − 106**		2.2547*E* − 106		7.9515*E* − 106		3.4630*E* − 98		1.6367*E* − 74		1.0385*E* − 60	
F12 mean	3.0928*E* − 05	**10**	2.−14	**6**	3.8303*E* − 16	**3**	**7.7723*E* − 17**	**1**	4.9165*E* − 16	**4**	1.2857*E* − 11	**7**
Std.	1.6940*E* − 04		1.1912*E* − 13		1.1343*E* − 15		**4.2566*E* − 16**		8.0839*E* − 16		7.0414*E* − 11	
F13 mean	2.0321*E* − 01	**5**	1.9654*E* − 01	**3**	1.8321*E* − 01	**2**	**1.1987*E* − 01**	**1**	1.9987*E* − 01	**4**	2.1987*E* − 01	**7**
Std.	3.1984*E* − 02		3.1984*E* − 02		3.7905*E* − 02		**4.0684*E* − 02**		2.6261*E* − 02		4.8423*E* − 02	
F14 mean	2.4212*E* − 01	**8**	2.4905*E* − 01	**9**	1.4753*E* − 01	**5**	1.0062*E* − 01	**2**	1.6718*E* − 01	**6**	1.1603*E* − 01	**3**
Std.	1.6847*E* − 01		1.9466*E* − 01		9.4435*E* − 02		3.3954*E* − 03		4.8375*E* − 02		1.1973*E* − 02	
F15 mean	**0.0000 *E* + 00**	**1**	0.0000 *E* + 00	**1**	**0.0000 *E* + 00**	**1**	**0.0000 *E* + 00**	**1**	2.3950*E* − 236	**2**	1.6645*E* − 187	**3**
Std.	**0.0000 *E* + 00**		0.0000 *E* + 00		**0.0000 *E* + 00**		**0.0000 *E* + 00**		0.0000 *E* + 00		0.0000 *E* + 00	
F16 mean	1.0914*E* − 12	**6**	8.7918*E* − 13	**5**	1.1141*E* − 12	**7**	4.3201*E* − 12	**8**	3.7138*E* − 13	**4**	3.3348*E* − 13	**3**
Std.	8.9447*E* − 13		1.0146*E* − 12		1.5263*E* − 12		1.9162*E* − 11		1.9333*E* − 13		1.2991*E* − 13	
F17 mean	5.1744 *E* + 05	**11**	3.4622 *E* + 05	**9**	4.0731 *E* + 05	**10**	8.0419 *E* + 05	**12**	1.5593 *E* + 05	**8**	8.4804 *E* + 04	**7**
Std.	2.8828 *E* + 05		1.3763 *E* + 05		2.0986 *E* + 05		4.5759 *E* + 05		1.0031 *E* + 05		6.3997 *E* + 04	
F18 mean	3.6167 *E* + 02	**12**	2.2199 *E* + 01	**11**	1.6293 *E* + 01	**10**	2.3579*E* − 01	**7**	5.5248 *E* + 00	**9**	2.7280 *E* + 00	**8**
Std.	3.4804 *E* + 02		2.3441 *E* + 01		2.0719 *E* + 01		2.9995*E* − 01		5.3507 *E* + 00		2.3433 *E* + 00	
F19 mean	8.8440 *E* + 01	**12**	8.1627*E* − 12	**3**	1.7751*E* − 09	**4**	6.2990*E* − 06	**8**	**6.0633*E* − 13**	**1**	3.6090*E* − 09	**6**
Std.	1.3947 *E* + 02		1.9885*E* − 11		9.6843*E* − 09		3.1457*E* − 05		**3.3022*E* − 13**		1.2103*E* − 08	
F20 mean	2.0909 *E* + 01	**3**	2.0923 *E* + 01	**6**	**2.0899 *E* + 01**	**1**	2.0908 *E* + 01	**2**	2.0921 *E* + 01	**5**	2.0926 *E* + 01	**7**
Std.	6.2772*E* − 02		4.8322*E* − 02		**6.6776*E* − 02**		5.5540*E* − 02		6.9368*E* − 02		4.6310*E* − 02	
F21 mean	2.3906 *E* + 01	**9**	2.5747 *E* + 01	**11**	2.4908 *E* + 01	**10**	2.8350 *E* + 01	**12**	2.1746 *E* + 01	**8**	2.0498 *E* + 01	**7**
Std.	2.8843 *E* + 00		3.0756 *E* + 00		2.7934 *E* + 00		2.9965 *E* + 00		3.2228 *E* + 00		2.6114 *E* + 00	
F22 mean	3.5454*E* − 01	**12**	3.0340*E* − 01	**10**	2.8817*E* − 01	**9**	3.0853*E* − 01	**11**	2.1249*E* − 01	**7**	1.1537*E* − 01	**5**
Std.	3.2317*E* − 01		1.7580*E* − 01		1.1671*E* − 01		1.3304*E* − 01		1.1696*E* − 01		7.6889*E* − 02	
F23 mean	3.7874 *E* + 03	**6**	3.3063 *E* + 03	**3**	3.6298 *E* + 03	**5**	3.3104 *E* + 03	**4**	**3.0790 *E*** + **03**	**1**	3.2067*E* + 03	**2**
Std.	8.3395 *E* + 02		7.4574 *E* + 02		7.2296 *E* + 02		5.8917 *E* + 02		**5.8848 *E*** + **02**		7.3814 *E* + 02	
F24 mean	1.1745 *E* + 01	**12**	1.1274 *E* + 01	**9**	1.1216 *E* + 01	**6**	1.1705 *E* + 01	**11**	1.1167 *E* + 01	**4**	1.1165 *E* + 01	**3**
Std.	4.9468*E* − 01		8.3977*E* − 01		6.8667*E* − 01		9.3060*E* − 01		8.5698*E* − 01		7.3902*E* − 01	
F25 mean	3.2821 *E* + 03	**8**	3.0343 *E* + 03	**7**	3.0077 *E* + 03	**5**	3.0111 *E* + 03	**6**	2.7380 *E* + 03	**2**	2.7457 *E* + 03	**3**
Std.	6.4796 *E* + 02		5.2848 *E* + 02		6.0257 *E* + 02		5.0123 *E* + 02		5.7139 *E* + 02		4.6850 *E* + 02	
F26 mean	2.2106 *E* + 03	**10**	2.0075 *E* + 03	**9**	2.8073 *E* + 03	**12**	2.7058 *E* + 03	**11**	9.3688 *E* + 02	**6**	**6.1365 *E* + 02**	**1**
Std.	9.2791 *E* + 02		7.0836 *E* + 02		2.5755 *E* + 03		1.6280 *E* + 03		2.7344 *E* + 02		**2.0362 *E* + 02**	
F27 mean	4.3187 *E* + 02	**11**	2.3164 *E* + 02	**9**	3.4622 *E* + 02	**10**	1.5558 *E* + 03	**12**	8.4483 *E* + 01	**8**	7.9338 *E* + 01	**7**
Std.	1.5688 *E* + 03		2.8944 *E* + 02		5.5363 *E* + 02		1.9408 *E* + 03		2.1385 *E* + 01		3.7933 *E* + 01	
F28 mean	1.6340 *E* + 02	**12**	1.2592 *E* + 02	**11**	1.1945*E* + 02	**10**	1.1183 *E* + 02	**9**	8.5297 *E* + 01	**8**	6.2142 *E* + 01	**7**
Std.	6.7125 *E* + 01		5.1143 *E* + 01		5.2491 *E* + 01		6.2047*E* + 01		4.1632 *E* + 01		1.9968 *E* + 01	
F29 mean	6.3684 *E* + 02	**9**	5.5887 *E* + 02	**6**	5.2171 *E* + 02	**4**	7.3378 *E* + 02	**12**	**4.1560 *E* + 02**	**1**	4.5805 *E* + 02	**2**
Std.	2.4983 *E* + 02		2.7218 *E* + 02		2.4827 *E* + 02		7.5234 *E* + 02		**1.6027 *E* + 02**		1.5578 *E* + 02	
F30 mean	2.1929*E* + 02	**7**	2.1535 *E* + 02	**2**	2.1836 *E* + 02	**6**	2.1757 *E* + 02	**5**	**2.1221 *E* + 02**	**1**	2.2536 *E* + 02	**10**
Std.	1.8484 *E* + 01		1.6550 *E* + 01		1.7093 *E* + 01		1.5568 *E* + 01		**1.3611 *E* + 01**		6.1665 *E* + 00	
**Number of winners**		**7**		**5**		**7**		**10**		**7**		**3**
F1 mean	1.8634*E* − 144	**4**	3.3710*E* − 130	**5**	6.6891*E* − 103	**6**	5.6670*E* − 91	**7**	7.4384*E* − 81	**8**	1.5166*E* − 74	**9**
Std.	7.8287*E* − 144		7.3291*E* − 130		2.6303*E* − 102		1.9990*E* − 90		3.2S044*E* − 80		4.9493*E* − 74	
F2 mean	1.0174*E* − 146	**4**	1.2462*E* − 131	**5**	8.2644*E* − 105	**6**	6.7337*E* − 93	**7**	5.3107*E* − 83	**8**	2.3385*E* − 76	**9**
Std.	2.2306*E* − 146		3.8761*E* − 131		2.8562*E* − 104		2.1117*E* − 92		1.3153*E* − 82		4.7131*E* − 76	
F3 mean	8.6727*E* − 27	**7**	2.6669*E* − 24	**8**	1.0175*E* − 17	**10**	8.7691*E* − 18	**9**	1.0958*E* − 17	**11**	1.4858*E* − 16	**12**
Std.	2.4801*E* − 26		1.2058*E* − 23		3.0450*E* − 17		1.5707*E* − 17		2.2461*E* − 17		2.9935*E* − 16	
F4 mean	1.9003*E* − 03	**6**	2.7789*E* − 03	**11**	3.6375*E* − 03	**12**	2.7137*E* − 03	**9**	2.0692*E* − 03	**8**	2.4249*E* − 03	**10**
Std.	7.0614*E* − 04		1.0254*E* − 03		1.2242*E* − 03		9.0594*E* − 04		6.1624*E* − 04		7.4433*E* − 04	
F5 mean	**0.0000 *E*** + **00**	**1**	3.0540*E* − 01	**2**	2.5139 *E* + 00	**7**	9.1928*E* − 01	**6**	6.5257*E* − 01	**5**	5.0356*E* − 01	**4**
Std.	**0.0000 *E*** + **00**		1.6727 *E* + 00		5.5399 *E* + 00		2.9102 *E* + 00		1.7325 *E* + 00		1.5684 *E* + 00	
F6 mean	7.2239*E* − 15	**4**	8.0528*E* − 15	**8**	7.5791*E* − 15	**6**	7.8160*E* − 15	**7**	7.5791*E* − 15	**6**	7.1054*E* − 15	**3**
Std.	1.4703*E* − 15		2.4567*E* − 15		1.8027*E* − 15		2.1681*E* − 15		1.8027*E* − 15		0.0000 *E* + 00	
F7 mean	**0.0000 *E*** + **00**	**1**	**0.0000 *E*** + **00**	**1**	**0.0000 *E*** + **00**	**1**	**0.0000 *E*** + **00**	**1**	**0.0000 *E*** + **00**	**1**	**0.0000 *E*** + **00**	**1**
Std.	**0.0000 *E*** + **00**		**0.0000 *E*** + **00**		**0.0000 *E*** + **00**		**0.0000 *E*** + **00**		**0.0000 *E*** + **00**		**0.0000 *E*** + **00**	
F8 mean	1.5547 *E* + 01	**4**	**1.3778 *E*** + **01**	**1**	1.7801 *E* + 01	**7**	1.6904 *E* + 01	**6**	1.5922 *E* + 01	**5**	1.4829 *E* + 01	**2**
Std.	1.6655 *E* + 00		**8.3997*E* − 01**		2.0629 *E* + 00		1.3511 *E* + 00		7.6778*E* − 01		7.3994*E* − 01	
F9 mean	1.3823*E* − 02	**2**	4.1464*E* − 02	**5**	6.9108*E* − 02	**7**	7.6016*E* − 02	**9**	2.4189*E* − 02	**3**	**1.0367*E* − 02**	**1**
Std.	3.5843*E* − 02		8.8627*E* − 02		9.1643*E* − 02		1.4893*E* − 01		5.2247*E* − 02		**3.1632*E* − 02**	
F10 mean	**0.0000 *E*** + **00**	**1**	**0.0000 *E*** + **00**	**1**	**0.0000 *E*** + **00**	**1**	**0.0000 *E*** + **00**	**1**	**0.0000 *E*** + **00**	**1**	**0.0000 *E*** + **00**	**1**
Std.	**0.0000 *E*** + **00**		**0.0000 *E*** + **00**		**0.0000 *E*** + **00**		**0.0000 *E*** + **00**		**0.0000 *E*** + **00**		**0.0000 *E*** + **00**	
F11 mean	5.6481*E* − 50	**7**	1.4373*E* − 44	**8**	4.9543*E* − 33	**9**	1.1272*E* − 31	**10**	3.6466*E* − 30	**11**	3.4290*E* − 28	**12**
Std.	1.8424*E* − 49		3.6834*E* − 44		1.2025*E* − 32		2.5961*E* − 31		4.7243*E* − 30		5.1504*E* − 28	
F12 mean	1.1665*E* − 16	**2**	3.1371*E* − 10	**8**	4.4620*E* − 04	**12**	3.9128*E* − 05	**11**	9.3514*E* − 08	**9**	1.7797*E* − 15	**5**
Std.	4.4445*E* − 16		1.7165*E* − 09		9.6886*E* − 04		2.0864*E* − 04		4.8628*E* − 07		1.6281*E* − 15	
F13 mean	2.0987*E* − 01	**6**	2.3987*E* − 01	**9**	2.7321*E* − 01	**11**	2.3989*E* − 01	**10**	2.3321*E* − 01	**8**	2.0987*E* − 01	**6**
Std.	3.0513*E* − 02		4.9827*E* − 02		5.8329*E* − 02		4.9812*E* − 02		4.7946*E* − 02		3.0513*E* − 02	
F14 mean	1.3266*E* − 01	**4**	1.7522*E* − 01	**7**	3.5749*E* − 01	**10**	4.2629*E* − 01	**11**	6.7110*E* − 01	**12**	**1.0031 *E*** + **00**	**1**
Std.	3.2946*E* − 02		5.7259*E* − 02		1.3949*E* − 01		2.4293*E* − 01		2.7434*E* − 01		**3.1508*E* − 01**	
F15 mean	6.2031*E* − 149	**4**	2.0046*E* − 134	**5**	8.7140*E* − 106	**6**	1.3911*E* − 94	**7**	4.8466*E* − 85	**8**	7.4000*E* − 79	**9**
Std.	1.4971*E* − 148		4.4859*E* − 134		3.1137*E* − 105		4.1234*E* − 94		1.3312*E* − 84		1.3354*E* − 78	
F16 mean	3.3348*E* − 13	**3**	2.5769*E* − 13	**2**	1.9115*E* − 08	**10**	1.7205*E* − 11	**9**	**2.3495*E* − 13**	**1**	**2.3495*E* − 13**	**1**
Std.	1.2991*E* − 13		7.8614*E* − 14		2.0880*E* − 08		3.7190*E* − 11		**4.1513*E* − 14**		**4.1513*E* − 14**	
F17 mean	2.5911 *E* + 04	**6**	2.0236 *E* + 04	**5**	1.5404 *E* + 04	**4**	4.2028*E* + 03	**3**	1.3939 *E* + 03	**2**	**3.9232 *E* + 02**	**1**
Std.	1.7876 *E* + 04		2.0596 *E* + 04		1.7468 *E* + 04		1.0755 *E* + 04		2.2990 *E* + 03		**5.2340 *E* + 02**	
F18 mean	8.3293*E* − 02	**6**	**2.0654*E* − 04**	**1**	1.0079*E* − 02	**2**	2.7159*E* − 02	**4**	3.3594*E* − 02	**5**	2.5218*E* − 02	**3**
Std.	1.5820*E* − 01		**2.1159*E* − 04**		3.6116*E* − 03		1.0117*E* − 02		1.0102*E* − 02		9.7995*E* − 03	
F19 mean	1.0383*E* − 12	**2**	1.9659*E* − 06	**7**	2.1229 *E* + 01	**11**	6.9545 *E* + 00	**10**	1.2045*E* − 05	**9**	3.3831*E* − 09	**5**
Std.	9.6454*E* − 13		6.9306*E* − 06		2.3423 *E* + 01		1.1080 *E* + 01		3.1678*E* − 05		5.1730*E* − 09	
F20 mean	2.0921 *E* + 01	**5**	2.0915 *E* + 01	**4**	2.0944 *E* + 01	**11**	2.0932 *E* + 01	**10**	2.0931 *E* + 01	**9**	2.0930 *E* + 01	**8**
Std.	4.9477*E* − 02		6.0050*E* − 02		3.8063*E* − 02		6.2609*E* − 02		6.4298*E* − 02		6.4638*E* − 02	
F21 mean	1.8475 *E* + 01	**5**	1.7112 *E* + 01	**4**	1.9149 *E* + 01	**6**	1.7047 *E* + 01	**2**	**1.6573 *E* + 01**	**1**	1.7062 *E* + 01	**3**
Std.	2.2045*E* + 00		3.1375 *E* + 00		3.0854 *E* + 00		2.2433 *E* + 00		**3.8705 *E* + 00**		4.7870 *E* + 00	
F22 mean	1.2080*E* − 01	**6**	7.6487*E* − 02	**4**	2.7264*E* − 01	**8**	4.9529*E* − 02	**2**	**4.6303*E* − 02**	**1**	5.7641*E* − 02	**3**
Std.	6.9533*E* − 02		5.9331*E* − 02		5.0913*E* − 01		3.4914*E* − 02		**2.4240*E* − 02**		4.5834*E* − 02	
F23 mean	3.8294 *E* + 03	**7**	4.0173 *E* + 03	**8**	4.7015 *E* + 03	**9**	5.0416 *E* + 03	**10**	5.2883 *E* + 03	**11**	5.5463 *E* + 03	**12**
Std.	7.4079 *E* + 02		7.2649 *E* + 02		9.3202 *E* + 02		7.7981 *E* + 02		4.3313 *E* + 02		3.8622 *E* + 02	
F24 mean	1.1178 *E* + 01	**5**	**1.1054 *E* + 01**	**1**	1.1128 *E* + 01	**2**	1.1231 *E* + 01	**7**	1.1235 *E* + 01	**8**	1.1365 *E* + 01	**10**
Std.	6.6333*E* − 01		**7.1771*E* − 01**		6.6137*E* − 01		4.7694*E* − 01		5.4140*E* − 01		5.2287*E* − 01	
F25 mean	**2.6819 *E* + 03**	**1**	2.8717 *E* + 03	**4**	3.4417 *E* + 03	**9**	3.3570 *E* + 03	**10**	3.6201 *E* + 03	**11**	4.4863 *E* + 03	**12**
Std.	**6.5599 *E* + 02**		6.5461 *E* + 02		8.6057 *E* + 02		7.3188 *E* + 02		8.4552 *E* + 02		6.6389 *E* + 02	
F26 mean	6.3444 *E* + 02	**2**	6.7682 *E* + 02	**3**	7.9835 *E* + 02	**4**	9.1618 *E* + 02	**5**	9.8952 *E* + 02	**7**	9.9537 *E* + 02	**8**
Std.	2.3050 *E* + 02		1.6475 *E* + 02		2.4100 *E* + 02		1.9385 *E* + 02		1.6113 *E* + 02		1.8164 *E* + 02	
F27 mean	**5.3847 *E* + 01**	**1**	5.8104 *E* + 01	**4**	6.1993*E* + 01	**5**	6.3941 *E* + 01	**6**	5.6147 *E* + 01	**2**	5.6436 *E* + 01	**3**
Std.	**1.6743 *E* + 01**		1.4715 *E* + 01		1.1871 *E* + 01		1.2469 *E* + 01		1.0674 *E* + 01		9.3082 *E* + 00	
F28 mean	4.1302 *E* + 01	**5**	4.3142 *E* + 01	**6**	3.7295 *E* + 01	**2**	3.8066 *E* + 01	**3**	3.8498 *E* + 01	**4**	**3.5921 *E* + 01**	**1**
Std.	1.5566 *E* + 01		1.6008 *E* + 01		1.2944 *E* + 01		6.7568 *E* + 00		6.7459 *E* + 00		**7.0100 *E* + 00**	
F29 mean	4.9136 *E* + 02	**3**	5.9505 *E* + 02	**7**	5.4938 *E* + 02	**5**	6.3168 *E* + 02	**8**	6.9930 *E* + 02	**11**	6.8864 *E* + 02	**10**
Std.	1.7069 *E* + 02		1.2566 *E* + 02		1.5177 *E* + 02		1.3670 *E* + 02		1.3562 *E* + 02		9.5989 *E* + 01	
F30 mean	2.1627 *E* + 02	**3**	2.2452 *E* + 02	**9**	2.2704 *E* + 02	**12**	2.2677 *E* + 02	**11**	2.2398 *E* + 02	**8**	2.1671 *E* + 02	**4**
Std.	1.3038 *E* + 01		9.7575 *E* + 00		1.0816 *E* + 01		5.2881 *E* + 00		7.4227 *E* + 00		1.1142 *E* + 01	
**Number of winners**		**5**		**5**		**2**		**2**		**5**		**7**

The article "An Evolutionary Frog Leaping Algorithm for Global Optimization Problems and Applications" was published in 2021. Journal: Comput Intell Neurosci.

**Table 14:** Friedman test for EFLAs.

Order	Algorithm	Averages ranks
**1**	**EFLA07**	**4.73**
2	EFLA05	5.02
3	EFLA03	5.62
4	EFLA06	5.90
5	EFLA08	6.05
6	EFLA02	6.28
7	EFLA04	6.35
8	EFLA12	6.83
9	EFLA11	7.40
10	EFLA01	7.72
11	EFLA09	8.05
12	EFLA10	8.05

**Table 15:** Statistical value of the Friedman test for EFLA.

Method	Statistical value	*p* value
Friedman test	34.493	3.00*E* − 4

**Table 16:** Comparison results for running times of 13 algorithms.

Algorithms	R_All	Friedman test (averages ranks)	F26	R	F27	R	F28	R	F29	R	F30	R
LAPO mean	**2**	2.00	18.85073	**2**	21.11916	**2**	**10.19375**	**1**	15.70117	**2**	26.02402	**3**
Std.			14.73749		8.33219		**5.046945**		5.138322		10.486	
TSQPSO mean	**7**	8.00	83.41357	**9**	73.35816	**8**	63.16787	**7**	62.40167	**5**	80.70665	**11**
Std.			31.49291		23.23443		38.22815		18.79341		22.89638	
WQPSO mean	**5**	7.20	72.62881	**4**	68.48122	**5**	54.22318	**5**	72.05188	**9**	94.39364	**13**
Std.			13.95612		15.88942		4.882538		16.00365		30.18515	
GbABC mean	**1**	**1.20**	**14.00864**	**1**	**13.3273**	**1**	23.13617	**2**	**13.57485**	**1**	**21.85513**	**1**
Std.			**1.927354**		**1.427645**		8.680884		**0.491732**		**2.723891**	
NNA mean	**8**	9.00	79.35531	**8**	70.78343	**7**	65.0304	**8**	85.66919	**13**	69.78715	**9**
Std.			25.49979		23.38431		28.41953		28.96784		59.49232	
SaDE mean	**11**	10.80	84.98572	**10**	84.29369	**11**	79.89936	**13**	80.65329	**12**	69.2513	**8**
Std.			19.33125		16.18581		31.65429		14.61335		23.55451	
SFLA mean	**6**	7.80	136.3891	**12**	125.1609	**12**	57.82334	**6**	67.01151	**7**	25.03748	**2**
Std.			40.36156		20.92804		13.48065		42.31711		2.74917	
SSA mean	**7**	8.00	73.86124	**6**	69.47877	**6**	67.93734	**10**	68.23441	**8**	75.2461	**10**
Std.			8.404463		6.302224		4.591637		5.122081		4.807183	
CMAES mean	**10**	9.40	146.7898	**13**	75.25055	**9**	73.71599	**12**	64.8051	**6**	62.04743	**6**
Std.			154.6333		8.397211		21.58189		10.05967		4.808734	
SCA mean	**8**	9.00	72.91107	**5**	74.07331	**10**	67.25726	**9**	78.53473	**10**	82.08589	**12**
Std.			8.772488		6.297513		4.347105		8.089436		7.584847	
AAA mean	**3**	3.20	42.31129	**3**	41.42464	**3**	52.36864	**3**	38.31735	**3**	48.02182	**4**
Std.			20.78658		12.95451		12.77487		8.288076		9.548955	
GWO mean	**9**	9.20	115.0754	**11**	146.3654	**13**	53.906	**4**	80.47329	**11**	66.43477	**7**
Std.			30.3304		20.57077		5.832788		4.622302		16.92118	
EFLA mean	**4**	6.20	77.65418	**7**	61.11634	**4**	69.18329	**11**	60.45171	**4**	61.77447	**5**
Std.			49.93137		17.75919		13.70716		14.07025		2.787357	

The article "An Evolutionary Frog Leaping Algorithm for Global Optimization Problems and Applications" was published in 2021. Journal: Comput Intell Neurosci.

**Table 17:** Parameters setting.

NO.	Algorithm	Parameter setting
1	LAPO	**pop_size** **=** **40**
2	TLBO	**pop_size** **=** **20**
3	LSHADE	p_best_rate = 0.11, arc_rate = 2.6, memory_size = 6, pop_size = 18 *∗* 2, min_pop_size = 4.0
4	LSHADE−cnEpSin	p_best_rate = 0.11, arc_rate = 1.4, memory_size = 5, pop_size = 18 *∗* 2, min_pop_size = 4.0
13	EFLA	*m* = 6, *n* = 5, **pop_size** **=** **30**

**Table 18:** Details of six data sets.

No.	Data set	Number of class	Dimension	Number of samples
F1	Glass	6	10	214
F2	Wine	3	14	178
F3	OBCW	2	10	699
F4	PBCW	2	33	198
F5	WDBC	2	31	569
F6	Heart	2	13	270

**Table 19:** Comparison with EFLA and 4 algorithms (LAPO, TLBO, LSHADE, and LSHADE-cnEpSin) for SVM.

	LAPO (%)	TLBO (%)	LSHADE (%)	LSHADE−cnEpSin (%)	EFLA (%)
F1 median	72.897	**74.766**	**74.766**	**74.766**	73.832
Std.	9.0204*e* − 001	1.4980*e* − 014	1.4777	1.9703*e* − 001	6.3013
F2 median	**98.876**	**98.876**	**98.876**	**98.876**	**98.876**
Std.	**2.9160*e* − 014**	1.4980*e* − 014	1.4980	2.3687*e* − 001	**2.9160*e* − 014**
F3 median	**96.853**	**96.853**	**96.853**	**96.853**	**96.853**
Std.	**3.1990*e* − 002**	7.5400*e* − 002	0	4.5240*e* − 002	**8.6524*e* − 002**
F4 median	82.323	82.323	82.323	82.323	**82.828**
Std.	0.00*e* + 000	0.00*e* + 000	0.00*e* + 000	0.00*e* + 000	**2.0727*e* − 001**
F5 median	**98.067**	**98.067**	**98.067**	**98.067**	**98.067**
Std.	**1.4580*e* − 014**	1.4980*e* − 014	1.6673	5.5576*e* − 002	**7.2125*e* − 002**
F6 median	69.259*e* + 001	69.630	68.889	69.259	**70.000**
Std.	3.0399*e* − 001	3.1232*e* − 001	3.1232*e* − 001	5.1793*e* − 001	**1.6454*e* − 001**

## Data Availability

The data used to support the results of this study are obtained from the corresponding author upon request.
